The article "A Comprehensive Survey on the Progress, Process, and Challenges of Lung Cancer Detection and Classification" was published in 2022. Journal: J Healthc Eng.

# A Comprehensive Survey on the Progress, Process, and Challenges of Lung Cancer Detection and Classification

**DOI:** 10.1155/2022/5905230

**Published:** 2022-12-16

**Authors:** M. F. Mridha, Akibur Rahman Prodeep, A. S. M. Morshedul Hoque, Md. Rashedul Islam, Aklima Akter Lima, Muhammad Mohsin Kabir, Md. Abdul Hamid, Yutaka Watanobe

**Affiliations:** ^1^Department of Computer Science and Engineering, American International University Bangladesh, Dhaka 1229, Bangladesh; ^2^Department of Computer Science and Engineering, Bangladesh University of Business and Technology, Dhaka 1216, Bangladesh; ^3^Department of Computer Science and Engineering, University of Asia Pacific, Dhaka 1216, Bangladesh; ^4^Department of Information Technology, King Abdulaziz University, Jeddah 21589, Saudi Arabia; ^5^Department of Computer Science and Engineering, University of Aizu, Aizuwakamatsu 965-8580, Japan

## Abstract

Lung cancer is the primary reason of cancer deaths worldwide, and the percentage of death rate is increasing step by step. There are chances of recovering from lung cancer by detecting it early. In any case, because the number of radiologists is limited and they have been working overtime, the increase in image data makes it hard for them to evaluate the images accurately. As a result, many researchers have come up with automated ways to predict the growth of cancer cells using medical imaging methods in a quick and accurate way. Previously, a lot of work was done on computer-aided detection (CADe) and computer-aided diagnosis (CADx) in computed tomography (CT) scan, magnetic resonance imaging (MRI), and X-ray with the goal of effective detection and segmentation of pulmonary nodule, as well as classifying nodules as malignant or benign. But still, no complete comprehensive review that includes all aspects of lung cancer has been done. In this paper, every aspect of lung cancer is discussed in detail, including datasets, image preprocessing, segmentation methods, optimal feature extraction and selection methods, evaluation measurement matrices, and classifiers. Finally, the study looks into several lung cancer-related issues with possible solutions.

## 1. Introduction

Lung cancer is a significant obstacle to the survival of humans, and many people lose their lives every year because of lung cancer. Early detection of pulmonary nodules is essential for improving lung cancer patients' survival rates. Nodules are abnormal tissue growths that can occur anywhere in the body. They can also grow in in-depth skin tissues as well as internal organs. When a nodule forms in the lungs, it is referred to as a pulmonary nodule. A nodule with a diameter of three centimeters or less is called a tumor [1]. There are mainly two kinds of tumors. It can be either malignant or benign. Malignant tumors mean cancerous tumors. It can grow and spread all over the body. On the other hand, benign tumors are not cancerous. They either do not spread or grow very slowly or do so. They usually do not return after being removed by a physician. Approximately 95% of lung nodules are benign [2]. But it can be malignant also. A larger lung nodule, such as 30 millimeters or more in diameter, has a higher risk of being cancerous than a smaller lung nodule [3].

The article "A Comprehensive Survey on the Progress, Process, and Challenges of Lung Cancer Detection and Classification" was published in 2022. Journal: J Healthc Eng.

Lung cancers are broadly divided into non-small-cell lung cancer (NSCLC) and small-cell lung cancer (SCLC) [4]. About 80%–85% of lung cancers are NSCLC, and 10%–15% of all lung cancers are SCLC. The survival rate of lung cancer is low. In 2008, there were 12.7 million cancer cases and 7.6 million cancer deaths, with 56% of patients and 64% of fatalities occurring in economically developing countries. Lung cancer is the most common cancer site in men, accounting for 17% of all new cancer cases and 23% of cancer deaths [5]. Lung cancer is diagnosed at an advanced stage in approximately 70% of patients, with a 5-year survival rate of approximately 16%. However, if lung cancer is detected early, it has a better chance of being treated successfully, with a 5-year survival rate of 70% [6, 7]. One of the leading causes of lung cancer is smoking. It can even happen to those who have never smoked. It can be increased by exposure to secondhand smoking, arsenic, asbestos, radioactive dust, or radon.

Several attempts have been made since 1980 to develop a system that can detect, segment [8, 9], and diagnose pulmonary nodules from CT scans [10]. The detection of pulmonary nodules is complicated because their appearance varies depending on their type, whether they are malignant, and their size, internal structure, and location. Segmentation has become a big problem, and it now requires a lot of different methods to solve it. Each technique focuses on another part of the problem [11]. These systems are referred to as computer-aided diagnosis systems (CAD). They go beyond simple image processing to provide specific information about the lesion that can aid radiologists in making a diagnosis. The idea of CAD was initially presented in 1966 [12]. Researchers first thought about using computers to make automated diagnoses. There were no other ideas or technologies at the time, so CAD technology was still in its infancy until the 1980s when the concept moved from automatic computer diagnosis to CAD [13]. The relevant ideas and computer technology were also quickly evolving at the time. All of these factors contributed to the advancement of CAD technologies. The first study on lung cancer CAD systems based on CT scans was published in 1991 [14]. Several competitions, such as Lung Nodule Analysis 2016 (LUNA16) [15] and Kaggle Data Science Bowl (KDSB) [16], have attracted several professional teams who have created lung cancer CAD algorithms in recent years. By making it easier to compare alternative algorithms, these competitions have aided in advancing lung cancer CAD technology. Lung cancer CAD can detect lung nodules and predict the likelihood of malignancy, making it a handy tool for doctors. Computer-aided detection (CADe) and computer-aided diagnosis (CADx) systems are two types of CAD systems. The former can detect and locate pulmonary nodules, while the latter can classify them as benign or malignant.

The article "A Comprehensive Survey on the Progress, Process, and Challenges of Lung Cancer Detection and Classification" was published in 2022. Journal: J Healthc Eng.

Several researchers analyzed the existing articles previously for detecting and diagnosing lung nodules using CT images. Yang et al. [17] examined the use of deep learning techniques to detect and diagnose lung nodules in particular. Convolutional neural networks (CNNs) have been the most widely used deep learning methods in treating pulmonary nodules. CNNs have produced excellent results in lung cancer CAD systems. In the 2017 DSB competition, for example, the winning team's algorithm was a CNN model [18], and a CNN model developed by Google and published in Nature outperformed six professional radiologists [19]. The problem of pulmonary nodule application has been tackled using various deep learning methods. Poap et al. [20] introduced a heuristic and nature-inspired method for X-ray image segmentation-based detection over aggregated images. The proposed approach for automating medical exams delivers favorable results for detecting diseased and healthy tissues. A heuristic red fox heuristic optimization algorithm (RFOA) was also presented for medical image segmentation by Jaszcz et al. [21]. In addition, the operation of heuristics was modified for the analysis of two-dimensional images, with an emphasis on equation modification and the development of a unique fitness function. Kumar et al. [22] were the first to employ an autoencoder (AE) to differentiate benign from malignant pulmonary nodules, while Chen et al. [23] were the first to use a deep belief network (DBN) in the context of pulmonary nodule CAD. To improve training efficiency, Wang and Chakraborty [24] proposed a sliced recurrent neural network (RNN) model. In their method, multiple layers of the RNN were taught simultaneously, which reduced training time. To train a deep learning model, a large amount of data is required. However, few labeled datasets are available for researchers due to the need for specialists and the time-consuming nature of the effort. A generative adversarial network (GAN) is based on the negative training paradigm and uses training to generate new images that are comparable to the original, which has piqued the interest of many medical imaging researchers [25]. Some researchers have chosen to generate lung nodule images with a GAN to increase the amount of data available [26]. Lung cancer detection has become more structured, making it more usable and reliable. This structure provides a basic workflow diagram for detecting lung cancer. However, the structure is not always the same, and there may be variations. When it comes to lung cancer detection, the process is divided into several steps, including collecting images or datasets, preprocessing the images, segmentation, feature extraction, feature selection and classification, and receiving the results.  Figure 1 depicts the method for detecting cancer in images.

- *Dataset*. Dataset collection is the initial step to starting the process. There are mainly 3 types of image datasets used for lung cancer detection: computed tomography (CT) scans, magnetic resonance imaging (MRI), and X-rays. CT scan images are mainly used because of their high sensitivity and low cost. Also, it is more available rather than MRI and X-ray. More about the dataset is discussed in Section 3.
- *Preprocessing*. Image preprocessing is used to improve the original image's quality and interpretability. The primary goal of CT image preprocessing is to remove noise, artifacts, and other irrelevant information from raw images, improve image quality, and detect relevant information.  Section 5 has a brief discussion about it.
- *Segmentation*. The segmentation of CT images is an important step in detecting lung nodules and recognizing lung cancer. Pulmonary segmentation's main goal is to separate the pulmonary parenchyma from other tissues and organs accurately. It uses preprocessed medical images to calculate the volume of lung parenchyma.  Section 6 discusses a variety of segmentation algorithms.
- *Feature Extraction*. The features of the segmented lung images are extracted and analyzed in this step. Feature extraction is a process in which a large amount of raw data is divided and reduced to more manageable groups after being initially collected. It makes the process a lot less complicated. Feature extraction methods are described in Section 7.
- *Feature Selection*. Feature selection identifies and isolates the most consistent, non-redundant, and relevant features in model construction. Feature selection is primarily used to improve predictive model performance while lowering modeling computational costs. It is also a way to make the classification result more accurate.  Section 8 describes the most commonly used feature selection methods.
- *Classification*. Classification is dividing a given set of data into groups of similar characteristics. It separates benign and malignant nodules based on the feature that has been selected. Well-known classification methods are discussed in Section 9.
- *Result*. Finally, the detection result of lung cancer shows us where the cancerous cell is in the lung. It is discussed in Section 10.

The article "A Comprehensive Survey on the Progress, Process, and Challenges of Lung Cancer Detection and Classification" was published in 2022. Journal: J Healthc Eng.

Figure 2 addresses the taxonomy of this survey. The lung nodule and cancer analysis were separated into two artificial intelligence plans applied in clinical imaging. This clinical imaging was divided into seven categories. We chose studies from various eras based on their popularity to conduct this survey. We upheld a systematic review methodology in this study, which will aid future researchers in determining the general skeleton of an artificial intelligence-based lung nodule and cancer analysis. This survey gives a reasonable perspective on ML and DL structures occupied with distinguishing lung cancer. This concentration likewise addresses the identification and characterization of lung nodules and malignant growth using imaging strategies. Finally, this survey coordinates a few open exploration challenges and opportunities for future scientists. We agree that this review serves as an essential guide for researchers who need to work with clinical image characterization using artificial intelligence-based lung nodules and cancer analysis while using various clinical images.  Table 1 shows a correlation between the existing surveys and our survey.  Table 2 provides a summary of recent surveys and reviews that have been conducted on various approaches for the detection, segmentation, and classification of lung cancer.

The survey discusses the findings of various related research work areas like nodule classification, nodule identification, lung cancer detection, lung cancer verification, and so on. While looking at the present challenges, this study generates suggestions and recommendations for further research works. The total contributions of the research are as follows:

- The article gives an intelligible review of detecting systems of lung nodules and cancer.
- The article inspects lung nodule and cancer-detecting procedures depending on the existing systems, datasets, image preprocessing, segmentation, feature extraction, and selection techniques. Further, the paper exploits the benefits and limitations of those systems.
- The article gives the procedures to detect lung nodules and cancer in a well-organized way.
- Finally, the survey adapts the present challenges of lung nodules and cancer detection systems, with further research on pathological diagnosis.

The article "A Comprehensive Survey on the Progress, Process, and Challenges of Lung Cancer Detection and Classification" was published in 2022. Journal: J Healthc Eng.

After going through this division, one should adapt how to get started with this topic.

The remaining sections of the paper are organized as follows. The methodology of the survey is described in Section 2. Various categorized datasets obtainable publicly are displayed in Section 3. Imaging modalities are briefly described in Section 4.  Section 5 describes the preprocessing algorithm of the image dataset of lung cancer and nodules.  Section 6 discusses the segmentation process and algorithms. Section 7 discusses the most commonly used algorithms for extracting features from CT scans, X-rays, and MRI images.  Section 8 discusses the most commonly used methods for feature selection. Section 9 discusses the well-known classification and detection algorithms. A comprehensive exploration of the performance for lung cancer and nodule detection is discussed in Section 10. The challenges faced most commonly while detecting lung nodules and cancer are explained with their possible solutions in Section 11. Lastly, the conclusion of this article is given in Section 12.

## 2. Survey Methodology

The survey is analyzed following a process developed by Kitchenham [40, 41] called systematic literature review (SLR). This article divides the SLR processes into three different parts: the planning phase, the conducting phase, and the reporting phase. In the subsequent sections, the steps are discussed in detail.

### 2.1. Planning the Review

This section discusses the planning for creating this review article in detail. The following topics are elaborated upon in the next section. The first is the research topic, the second includes the review materials' sources, and the third includes the inclusion and exclusion criteria.

#### 2.1.1. Research Questions

The basic research questions were as follows:

1. RQ1: what is the importance of lung cancer detection?
2. RQ2: what type of image modalities is used for lung cancer detection?
3. RQ3: which datasets are usually used in lung cancer detection?
4. RQ4: what are the most used algorithms for feature selection and extraction, segmentation, classification, and detection?
5. RQ5: which evaluation matrices are used for lung cancer detection to evaluate the system?
6. RQ5: what are the current challenges and limitations of the existing research and the scope of potential future research for lung cancer detection?

#### 2.1.2. Source of Review Materials

The survey only looks at high-quality academic articles from MDPI, ScienceDirect, SpringerLink, IEEE Xplore, Hindawi, ACM Digital Library, etc. and papers from well-known conferences.

The article "A Comprehensive Survey on the Progress, Process, and Challenges of Lung Cancer Detection and Classification" was published in 2022. Journal: J Healthc Eng.

#### 2.1.3. Inclusion and Exclusion Criteria

The most important information for this survey is collected using PRISMA (Preferred Reporting Items for Systematic Reviews and Meta-Analyses), which is shown in Figure 3.  Table 3 shows the criteria that PRISMA uses to choose which studies to include and which ones to leave out. In addition, this table shows how to select a paper based on certain criteria and standards, which criteria are used, and whether the article is initially accepted or rejected.

### 2.2. Conducting the Review

This section explains how the necessary information is extracted from the articles. Five subphases are addressed to get the most important information and conduct a structured literature review.

#### 2.2.1. Topical Relationship

This section describes how the articles selected for this survey connect to the others.  Figure 4 shows a word cloud comprised of the papers' keywords and the most important terms from their titles. It indicates how closely the selected articles are connected.

#### 2.2.2. Aims and Outcomes

Objectives, contributions, and challenges of different useful articles are presented in Sections 1 and 11.

#### 2.2.3. Evaluation Metrics

All the evaluation matrices used for evaluation are explained in Section 10.

#### 2.2.4. Research Type

It indicates the type of documents, such as an academic journal, conference or workshop proceeding, book chapter, or thesis.

#### 2.2.5. Publication Year and Type

At the start of this project, 610 papers were gathered from different sources, and 423 were chosen for the survey. More than 90% of these articles were published between 2010 and 2021. Therefore, we used more recent articles to update this review.

### 2.3. Outcome

Finally, the obtained information is examined, existing issues and difficulties are addressed, and future research opportunities are presented.

## 3. Dataset

There are many frequently used datasets that researchers use for lung cancer diagnosis. From Table 4, it can be seen that the CT scan is currently the most reliable method for gathering data on nodule detection in lung cancer. X-rays and MRIs are also used to detect lung cancer and nodules. CT scan is used because it is a confined method that can handle most datasets well. CT scans provide a comprehensive approach for storing data for various reasons. First, the information must be procured and put away by some members or patients. It is unacceptable to have the same storing plan for different patients to get data. After the patients are prepared, individuals have to lie down on a table and go through a passage-like machine that will catch and gauge data. For some time, this data collection strategy has been in place, with a specific recording period dictated by the work's motivation. The data saved in these sessions and recordings are primarily lung nodule images estimated by blocks established in CT scans, X-rays, or MRI. CT scans, X-rays, or MRIs differ from one member to the next and from one session to the next. In this segment, the datasets are portrayed, just as the subjects and X-ray cylinder, indicators, and sessions.

The article "A Comprehensive Survey on the Progress, Process, and Challenges of Lung Cancer Detection and Classification" was published in 2022. Journal: J Healthc Eng.

## 4. Imaging Modalities

Imaging is vital for the analysis and treatment of lung nodules and cancer. Hence, this research exhibits that lung cancer analysis relies upon seven particular classifications of clinical imaging modalities. CT scan, Xray, MRI, ultrasound (US), positron emission tomography (PET) scan, and single-photon emission computed tomography (SPECT) are the seven clinical imaging modalities, and their combination is known as multimodalities. The CT scan is the most basic and widely used imaging modality in lung imaging. As per Table 4, most of the work was done in computed tomography (CT) scan images. The second-highest number of studies delivered is for X-ray images and MRI [103–106]. Another imaging technique known as a chest radiograph is an expensive method with limited accessibility. These should be the reasons for the lower adaptivity of chest radiographs in research, as this imaging strategy was used in a small number of examinations [107, 108]. Ultrasound (US) and PET scan imaging strategies were utilized distinctly in a couple of studies [109–111]. The SPECT imaging strategy has acquired prevalence as of late in lung nodule classification and malignant growth recognition. Because the thermogram dataset is not publicly available, a couple of studies used this imaging strategy [112]. Unfortunately, none of the researchers used histopathology. The well-known imaging strategies are depicted in greater detail in the following section.

### 4.1. X-Ray

A type of high-energy radiation, like electromagnetic waves, is called X-ray. An X-ray is also called X-radiation. X-ray imaging makes images of the inside of the human body. It shows the parts of the body in different shades of black and white [113]. The soft tissues in the human body, such as blood, skin, and muscle, absorb the majority of the X-ray and allow it to transit, resulting in dark gray areas on the film. However, a bone or tumor, which is thicker than soft tissue, prevents most X-rays from passing through and appears white on the film [104]. Gavelli and Giampalma [114] used X-ray images to detect lung cancer. They calculate the sensitivity and specificity for evaluating the outcome.

The article "A Comprehensive Survey on the Progress, Process, and Challenges of Lung Cancer Detection and Classification" was published in 2022. Journal: J Healthc Eng.

### 4.2. CT Scan

A computed tomography (CT) scan is a medical imaging method utilized in radiology to get comprehensive body images for diagnostic purposes. It merges a series of X-rays taken from various viewpoints around the body and makes cuts on the bones, veins, and delicate tissues inside the body [115]. CT scans point out a cross section of the body part like bones, organs, and soft tissues more clearly than standard X-rays because normal X-rays are done in two directions. It depicts the structure, size, and location of a tumor [116]. CT scans are more detailed than standard X-rays in identifying cross sections of body parts such as bones, organs, and delicate tissues [117]. In 2018, Makaju et al. [51] used CT scan images to detect lung cancer. Using their proposed model, they attempted to achieve 100% accuracy. Zheng et al. [118] also used CT images to detect lung cancer and inflammatory pseudo-tumor.

### 4.3. Magnetic Resonance Imaging (MRI)

MRI is a clinical imaging technique that utilizes radiofrequency signals to create point-by-point images of the organs and tissues in the body. MRI scanners use solid magnetic fields, magnetic field gradients, and radio waves to generate images of the organs in the body [119]. MRI creates images of soft tissues in the human body that are often difficult to see with other imaging techniques. As a result, it is highly effective at detecting and locating cancers. It also generates images that allow specialists to see the location of a lung tumor and estimate its shape and size. A specific dye named a contrast medium is applied to create a better image before the scan [106]. Cervino et al. [120] tried to track lung tumors by performing ANN in MRI sagittal images. The mean error was 7.2 mm using only TM and 1.7 mm when the surrogate was combined with TM.

### 4.4. Positron Emission Tomography (PET) Scan

PET scan is a helpful imaging method that uses radioactive substances known as radiotracers to envision and measure changes in metabolic cycles and other physiological activities, including circulation system, regional compound course of action, and absorption [121]. In addition, PET scan is a diagnostic tool that helps doctors detect cancer in the body. The scan employs a unique shading technique that includes radioactive tracers. Depending on which part of the body is being examined, these tracers are either swallowed, ingested, or implanted into a vein in the arm [122]. The PET scan utilizes a mildly radioactive medication to appear in spaces of the body where cells are more dynamic than regular cells. It is used to assist with diagnosing a few conditions, including malignant growth [123]. It can also help determine where the cancer has spread and whether or not it has spread. Because malignant growth cells have a higher metabolic rate than normal cells, they appear as bright spots on PET scans. Lung cancer is the bright spot in the chest that can be seen best on PET and PET-CT images [124]. Weder et al. [111] tried their model in PET scan and got a positive predictive value of 96%.

The article "A Comprehensive Survey on the Progress, Process, and Challenges of Lung Cancer Detection and Classification" was published in 2022. Journal: J Healthc Eng.

### 4.5. Single-Photon Emission Computed Tomography (SPECT)

SPECT is an atomic medication tomographic imaging method utilizing gamma rays. It is similar to traditional nuclear medicine planar imaging with a gamma camera, but it can provide accurate 3D data. However, it can provide accurate 3D data [125]. A SPECT scan is a test that shows how bloodstreams connect to tissues and organs [126]. Antibodies (proteins that recognize and adhere to cancer cells) can be linked to radioactive substances. First, assuming a tumor is available, the antibodies will be attached to it. Then, at that point, a SPECT output should be possible to recognize the radioactive substance and uncover where the cancer is found [127].

### 4.6. Multiple Modalities

Multiple modalities are considered an educational approach used to relieve the stress of researchers [128]. It entails giving various introductions and experiences of the substance to utilize multiple senses and abilities in a single example. Numerous modalities frequently cater to different learning styles [129]. Modalities can be performed using a combination of chemotherapy and radiation therapy. Concurrent chemoradiotherapy is the simultaneous administration of chemotherapy and radiation therapy [130]. Farjah et al. [131] implemented single, double, and tri-modality in their research. They conducted a CT scan for single modality, CT scan or PET scan with invasive staging for bi-modality, CT scan, PET Scan, and invasive stage for tri-modality.

The advantages and disadvantages of these image modalities are described in Table 5.

## 5. Image Preprocessing

Image preprocessing organizes images before they are used in model preparation and induction. The goal of preprocessing is to improve the quality of the image so that it can be investigated more thoroughly [132]. It includes, but is not limited to, rectifications for resizing, arranging, and shading [133]. As a result, in some cases, a change that could be an expansion may be better served as a preprocessing step in others.

### 5.1. Histogram Equalization

There are two different ways to contemplate and carry out histogram leveling, either as picture change or as range change [134]. Much of the time range change is preferable because it protects the initial data [135]. It is employed in image analysis. To produce a high contrast image, the gray level intensities are expanded along the *x*-axis [136]. Asuntha and Srinivasan [137] used a histogram evening out to close the gap. Shakeel et al. [90] changed differences in their dataset. Ausawalaithong et al. [98] preprocessed their picture dataset with histogram balance. It enhances the CT scan's contrast; it spreads out the most frequent pixel intensity values or stretches out the intensity range of the scan. Let *I* be a given CT scan image represented as a *I*_*x*_ by *I*_*y*_ matrix of integer pixel intensities ranging from 0 to 256. Let *N* denote the normalized histogram bin of image *I* for available intensity.

(1) $$\begin{array}{c} I_{N}=\frac{\text{number of pixels with available intensity }n}{\text{total number of pixels}}\text{,} \end{array}$$

where *n*=0,1,…, 255.

The article "A Comprehensive Survey on the Progress, Process, and Challenges of Lung Cancer Detection and Classification" was published in 2022. Journal: J Healthc Eng.

### 5.2. Median Filter Mask

The median filter is a non-straight computerized separating strategy, regularly used to eliminate roughness from an image or sign [138]. This type of noise reduction is a common prehandling step used to work on the aftereffects of later preparation. The median filter is a sifting procedure used to remove noise from images and signals [139]. The median filter is essential in image processing because it protects edges during clamor expulsion. It is broadly utilized as it is best at eliminating commotion while safeguarding borders [140]. Tun and Soe [141] used and claimed the median filter mask to be the best filter for their research. Shakeel et al. [142] and Ausawalaithong et al. [98] used a median filter mask in preprocessing their dataset. Asuntha and Srinivasan [137] reshaped and resized their data with a median filter. Sangamithraa and Govindaraju [143] used the median filter mask in image preprocessing to detect lung nodules. It moves through the lung images pixel by pixel, replacing each value with the median value of neighboring pixels. It can save sensitive components in a picture while filtering noise, and it is good at eliminating “salt and pepper” type noise.

### 5.3. Gaussian Filter

A Gaussian filter is a filter whose response is based on a Gaussian capacity [144]. This effect is widely used in design software, usually to smooth out images and reduce detail [145]. Gaussian noise, also known as Gaussian distribution, is a factual noise with a possible thickness equivalent to ordinary conveyance. This roughness is produced by combining irregular Gaussian capacity with image capacity [146]. This roughness can be eliminated by using a linear filter, as it is an ideal way of eliminating Gaussian roughness. Riquelme and Akhloufi [31], Teramoto et al. [147], and Rossetto and Zhou [148] used Gaussian filters to preprocess their image dataset. Ausawalaithong et al. [98], Hosny et al. [149], and Shakeel et al. [150] also utilized this filter to reshape their dataset and use those from detecting lung nodules. Al-Tarawneh [151] and Avanzo et al. [152] used CT scans and preprocessed them with the Gaussian filter. Asuntha et al. [153], Wang et al. [154], Sang et al. [65], and Ozdemir et al. [42] smoothed and preserved edges with the Gaussian filter. Fang [155] and Song et al. [156] applied the Gaussian filter on the LUNA16 [15] dataset to detect lung cancer. The effect of Gaussian smoothing is to blur CT scans of the lung similar to the mean filter. The standard deviation of the Gaussian determines the degree of smoothing. Gaussian blurring the CT image minimizes the amount of noise and reduces speckles.

(i) In 1D:
  (2) $$\begin{array}{c} g_{\sigma }\left(x\right)=\frac{1}{\sqrt{2\pi \sigma }}\exp\;\left(-\frac{x^{2}}{2\sigma^{2}}\right)\text{.} \end{array}$$
(ii) In 2D:
  (3) $$\begin{array}{c} G_{\sigma }\left(x,y\right)=\frac{1}{2\pi \sigma^{2}}\exp\;\left(-\frac{x^{2}+y^{2}}{2\sigma^{2}}\right)\text{,} \end{array}$$
where *σ* is referred to as standard deviation of the distribution. The mean of the distribution is considered as 0.

The article "A Comprehensive Survey on the Progress, Process, and Challenges of Lung Cancer Detection and Classification" was published in 2022. Journal: J Healthc Eng.

### 5.4. Wiener Filter

The Wiener filter is the MSE-ideal fixed straight filter for images corrupted by added substance clamor and obscuring. Wiener filter works when the sign and roughness measures are assumed to be fixed [157]. Sangamithraa and Govindaraju [143] removed the added substance noise while also modifying the obscuring. In terms of the mean square error, Wiener filtering is ideal.It is used to measure a perfect or arbitrary target interaction by straight time-invariant sifting of a detected noisy cycle, expecting to know fixed sign and noise spectra, and adding substance noise. [158]. It restricts the overall mean square error during backward sifting and commotion smoothing. It removes the additive noise and inverts the blurring simultaneously in lung images. It eliminates the additive noise, transforms the obscuring, and limits the general mean square error during inverse filtering and noise smoothing. The Wiener sifting is a direct assessment of the first picture [159].

### 5.5. Gabor Filter

A Gabor filter is a straight filter used in image processing for surface analysis, which means it determines whether or not there is a specific recurrence content in the lung images in explicit terms in a restricted district surrounding the point or region of examination [160]. It investigates whether there is a particular recurrence content. It has gotten significant consideration as it takes after the human visual framework. It is a neighborhood operation in which the value of any given pixel in the output lung scan is determined by applying some algorithm to the importance of the pixels in the neighborhood of the corresponding input pixel. To remove noise from the dataset, Mary and Dharma [161] used the Gabor filter.

(4) $$\begin{array}{c} F\left(u_{1},u_{2}\right)=\exp\;\left(-\frac{\left({\hat{u}}_{1}^{2}+\gamma^{2}{\hat{u}}_{2}^{2}\right)}{2\sigma^{2}}\right)\times \cos\;\left(\frac{2\pi }{\lambda }\hat{u_{1}}\right)\text{,}\\ \hat{u_{1}}=u_{1}\cos\;\theta +u_{2}\sin\;\theta \text{,}\\ \hat{u_{w_{2}}}=-u_{1}\sin\;\theta +u_{2}\cos\;\theta \text{,} \end{array}$$

where *λ* means the wavelength of the sinusoidal factor, *θ* represents the orientation of the normal to the parallel stripes of a Gabor function, *σ* is the sigma/standard deviation of the Gaussian envelope, and *γ* is the spatial aspect ratio and specifies the ellipticity of the support of the Gabor function.

The article "A Comprehensive Survey on the Progress, Process, and Challenges of Lung Cancer Detection and Classification" was published in 2022. Journal: J Healthc Eng.

### 5.6. Isotropic Voxel

Voxel is short for volume pixel, the littlest recognizable box-formed piece of a 3D picture. It could be compared to the 2D pixel [162]. The voxel size on CBCT images is isotropic, meaning that all sides are of the same size and have a uniform goal in every direction. The voxel technique was used by Nagao et al. [163] and Wang et al. [164] to reduce sharp noises and classify lung cancer. This method was also used by Quattrocchi et al. [165] to reshape their dataset to detect breast cancer and lung cancer.

### 5.7. Thresholding

Thresholding is a non-linear operation that changes a grayscale image into a binary image in which the two levels are allocated to pixels that are either below or above the set threshold value. It mainly converts an image from shading or grayscale into a twofold picture [166]. Thresholding is used to convert a low-contrast lung scan to a high-contrast lung scan. Thresholding is also a very effective tool in image segmentation. Its purpose is to convert grayscale images to binary format [151]. It takes the colorful or grayscale lung scans and turns them into binary scans. It diminishes the intricacy, works on acknowledgment and grouping, and changes the pixels to simplify the picture.

### 5.8. Binary Inversion

High-contrast picture reversal is a picture handling strategy where light regions are planned to dim, and dull areas are scheduled to light. A rearranged high-contrast picture can be considered an advanced negative of the first picture. Sharma et al. [167] used binary inversion to reduce noise from image datasets.

### 5.9. Interpolation

Image interpolation happens when one resizes or contorts one's image, starting with a one-pixel grid and then onto the next. Zooming refers to increasing the number of pixels in an image so that the image's details can be seen more clearly [168]. Interpolation is a well-known method for surveying dark characteristics that lie between known characteristics [169]. Interpolation is a course of deciding the obscure qualities in the middle of the realized information focus. It smooths, enlarges, or averages CT scans displayed with more pixels than that for which they have initially been reconstructed. It is used to foresee obscure qualities. It forecasts values for cubic in a raster. It is generally used to foresee the obscure qualities of any geological information, such as commotion level, precipitation, rise, and so on. The most common way to use test points with known qualities to figure out prices at other unknown issues is by insertion [170]. It could be used to predict dark characteristics for any geographic point data, such as height, precipitation, substance obsessions, disturbance levels, and so on [171]. Several insertion strategies have previously been reported. The broadly utilized strategies are the nearest neighbor, bilinear, bicubic, b-splines, lanczos2, and discrete wavelet transform. Lehmann et al. [172] and Zhao et al. [173] used interpolation in their dataset to detect nodules in the lungs. Liu et al. [58] used interpolation in CT scans and cleared noise, and Cascio et al. [174] used interpolation in 3D images to reduce noise.

The article "A Comprehensive Survey on the Progress, Process, and Challenges of Lung Cancer Detection and Classification" was published in 2022. Journal: J Healthc Eng.

### 5.10. Synthetic Minority Oversampling Technique (SMOTE)

SMOTE is an oversampling procedure that permits us to produce manufactured examples for our minority classes [175]. It is an oversampling method that creates fabricated models for the minority class. This computation aids in overcoming the overfitting problem caused by unpredictability in oversampling [176]. The imbalanced arrangement has the disadvantage of having too few instances of the minority class for a model to become comfortable with the choice limit [177]. Oversampling models from the minority class are regarded as one solution to this problem [178]. It randomly chooses a minority class instance and finds its *k* nearest minority class neighbors. The fabricated occasion is then created by arbitrarily selecting one of the *k* nearest neighbors *b* and coupling *a* and *b* to frame a line segment in the component space. The manufactured examples are made by mixing the two chosen occurrences, *a* and *b* [179]. While restructuring the information with SMOTE, Chen and Wu [180] found the risk factors. Patil et al. [181] utilized it to smooth textures and minimize noise. Wang et al. [182] employed SMOTE to remove borderlines.

The article "A Comprehensive Survey on the Progress, Process, and Challenges of Lung Cancer Detection and Classification" was published in 2022. Journal: J Healthc Eng.

### 5.11. Contrast Limited Adaptive Histogram Equalization (CLAHE)

Contrast limited AHE (CLAHE) is a variation of versatile histogram in which the differentiation enhancement is restricted to diminish this issue of clamor intensification [183]. It is utilized further to develop hazy pictures or video ability levels. It works on little districts in images, called tiles. The adjacent tiles are then consolidated using bi-linear insertion to remove the erroneous limits [184]. CLAHE calculation differs from standard HE in that CLAHE works on small areas of the image called tiles and registers a few histograms, each comparing to a specific segment of the image and using them to rearrange the advantages of the picture [185]. In CLAHE, the differentiation enhancement near given pixel value is provided by the incline of the change work [186]. Punithavathy et al. [187], Bhagyarekha and Pise [188], and Wajid et al. [189] used CLAHE as image preprocessing methodology. Technically, CLAHE does this by setting a threshold. If some gray levels in the lung scan exceed the threshold, the excess is evenly distributed to all gray levels. After this processing, the lung scan will not be over-enhanced, and the problem of noise amplification can be reduced.

Table 6 shows the pros and cons of these image preprocessing techniques.

## 6. Segmentation

Lung nodule segmentation is a crucial process designed to make the quantitative assessment of clinical criteria such as size, shape, location, density, texture, and the CAD system more manageable and more efficient [196–198]. However, because of their solidity, location, or texture, lung nodules such as juxta-pleural (nodules directly attached to the pleura's surface), juxta-vascular (nodules connected to vessels), and ground-glass nodules can be challenging to remove. Deep learning-based segmentation is a pixel-by-pixel categorization technique used to calculate organ probability [30]. This method is divided into two stages: the first is the creation of the probability map using CNN and image patches and the second is the refinement of the probability map using the general background of images and the probability map [196].

### 6.1. Watershed

Watershed segmentation is a technique for segmenting watersheds that use image morphology [199]. It requires the selection of at least one marker (“seed” point) within each image object, including the background as a separate object. The markers are picked by an operator or provided by an automatic mechanism that considers the object's application-specific information. A morphological watershed transformation helps to grow them after marking the items [200]. After the lung image preprocessing, noise is removed, images are smooth, and features are enhanced. Watershed is used in lung segmentation to identify the various regional maxima and minima [201].

The article "A Comprehensive Survey on the Progress, Process, and Challenges of Lung Cancer Detection and Classification" was published in 2022. Journal: J Healthc Eng.

### 6.2. U-Net

The U-Net [202] architecture is the most used architecture for medical image segmentation, and it significantly improves process performance. The fundamental parts of the U-Net are association of convolution layers in the contracting path and deconvolution layers in the expansive direction. It includes a contraction method for capturing anatomical structure and an asymmetrical expansion method for precise localization [28]. U-Net has enabled the segmentation process to form a spatial context at several scales despite the challenges of collecting both global and local contexts. As a result, it may be trained from end to end using only a small quantity of training data [28]. Convolution layers with rectified linear units and max-pooling layers make up the contracting route, similar to the classic architecture of a convolutional neural network. On the other hand, the expanding method entails sampling the feature map, followed by up-convolution and convolution layers using ReLU. Because of the loss of border pixels at each convolution, the extracting path's matching feature map must be cropped and concatenated with equivalent layers in the expensive direction [53]. The input photos and their respective masks are utilized for training the U-Net during the training phase. A lung image is supplied as input to generate the appropriate mask output during the testing phase. The mask is then applied to the relevant image to segment the area of interest, in this case, lung parenchyma [202].

### 6.3. Multiview Deep Convolutional Neural Network (MV-CNN)

The multiview deep convolutional neural network (MV-CNN) [203] architecture for lung nodule segmentation is a CNN-based architecture that proposes to transform lung nodule segmentation into CT voxel classification. The MV-CNN comprises three branches that process voxel patches from CT images in axial, coronal, and sagittal views. To obtain the voxel label, the three branches all have identical structures, including six convolutional layers, two max-pooling layers, and one fully connected layer. In addition, a parametric rectified linear unit (PReLU) [204] is implemented as a non-linear activation function after each convolutional layer and the first fully connected layer, and batch normalization is used for training acceleration [205].

### 6.4. Central Focused Convolutional Neural Network (CF-CNN)

The central focused convolutional neural network (CFCNN) [206] architecture includes three-dimensional and two-dimensional CT imaging views for lung nodules and cancer segmentation. It uses a CT image to extract a three-dimensional patch and a two-dimensional different plate patch self-contained on a single voxel as input to the CNN [207] model, which predicts whether the voxel belongs to the nodule or healthy tissue class. After feeding all voxels into this CNN model, a probability map assigns each voxel a probability of belonging to a nodule.

The article "A Comprehensive Survey on the Progress, Process, and Challenges of Lung Cancer Detection and Classification" was published in 2022. Journal: J Healthc Eng.

### 6.5. Fuzzy C-Means (FCM)

The FCM algorithm [208] is one of the most extensively used fuzzy clustering methods. Data elements can belong to multiple clusters in fuzzy clustering, and each part has a set of membership levels associated with it. It uses a CT image to extract a three-dimensional patch and a two-dimensional different plate patch self-contained on a single voxel as input to the CNN [207] model, which predicts whether the voxel belongs to the nodule or healthy tissue class. After feeding all voxels into this CNN model, a probability map assigns each voxel a probability of belonging to a nodule.

### 6.6. Hessian-Based Approaches

Image enhancement is performed on voxels in Hessian-based strategies to acquire the 3D Hessian matrix for each voxel and calculate the relevant eigenvalues. These eigenvalues are used to locate and segment lung nodules in a subsequent step. To begin, multiscale smoothing is used to reduce noise in the image and make nodule segmentation easier. Following that, the 3D Hessian matrix and associated eigenvalues are computed, and the results of each method are combined to produce the segmentation masks [209].

### 6.7. SegNet + Shape Driven Level Set

SegNet [210], a deep, fully convolutional network architecture, is used for coarse segmentation because it is designed primarily for pixelwise semantic labeling. A high-level network model SegNet is a network composed of encoders and decoders. SegNet is a preconfigured segmentation solution for a variety of medical imaging applications [211, 212]. A batch of lung field images is used during the training phase to feed the deep network. The output of CNN is used to initialize the level set function for lung nodule segmentation. The authors [213] used shape information as the primary image feature to guide the evolving shape to the intended item border.

### 6.8. Faster R-CNN

Faster R-CNN [214] is an improvement on the previous Fast R-CNN [215]. As the name implies, Faster R-CNN is much faster than Fast R-CNN due to the region proposal network (RPN). The model comprises two parts: the RPN and the Fast R-CNN. The input image is first subjected to convolution and pooling operations via the basic feature extraction network to obtain the image's feature map. After that, the feature map is transmitted to the RPN network, which performs preliminary border regression and classification judgment on the image. As the foundation for categorizing, the candidate frame is classified based on the background or object to be recognized. The RPN outputs the candidate frame's position and score information, and then they are sent to the Fast R-CNN for final processing by the fully connected layer. They are the final regression of the frame and the specific categorization of the object to be recognized in the final regression. First, ConvNet [216] is used to extract feature maps from lung pictures. Next, these are fed into RPN, which returns the candidate bounding boxes. The ROI pooling layer is then applied to reduce the size of the candidates. Finally, the proposals are transferred to a fully linked layer to obtain the final lung segmentation result [217].

The article "A Comprehensive Survey on the Progress, Process, and Challenges of Lung Cancer Detection and Classification" was published in 2022. Journal: J Healthc Eng.

### 6.9. Mask R-CNN

Mask R-CNN [80] is a compact and adaptable generic object instance segmentation system. It recognizes targets in images and provides high-quality segmentation results for each target. Mask R-CNN is divided into two sections, the first of which is RPN. It is a new network developed by Faster R-CNN [214] that replaces the previous R-CNN's selective search approach [215], and Fast R-CNN [215] integrates all content into a single network, significantly improving detection speed. The second stage features two concurrent branches, one for detection and the other for classification and bounding box regression. The mask branch is used for segmentation. The preprocessing program receives raw lung image sequences and generates 2D images before processing basic images such as coordinate transformation, slice selection, mask generation, and normalization. Then, it is used in the detection and segmentation module to detect and segment the locations and contours of expected pulmonary nodules [218].

### 6.10. Robust Active Shape Model (RASM)

Biomedical photos typically feature complicated objects that fluctuate significantly in appearance from one image to the next. It can be challenging to measure or recognize the existence of specific structures in such photos. The RASM [219] is trained using hand-drawn contours in training images. It employs principal component analysis (PCA) to identify critical variances in the training data, allowing the model to automatically determine whether a contour is a potentially excellent object contour [220, 221]. It also includes matrices that describe the texture of lines perpendicular to the control point; these are utilized to rectify positions during the search stage. The contour is deformed by finding the best texture match for the control points when the RASM is created. The movement of the control points is limited by what the RASM perceives as a “normal” object contour based on the training data in this iterative procedure. Then, PCA determines the formation's mean appearance (intensities) and variances in the training set. For example, the outline of the lungs is approximately segmented from lung images using a robust active shape model matching technique [222].

The article "A Comprehensive Survey on the Progress, Process, and Challenges of Lung Cancer Detection and Classification" was published in 2022. Journal: J Healthc Eng.

### 6.11. Region Growing

Growing a region is a bottom-up process that starts with a set of seed pixels [223]. The goal is for each seed to establish a uniformly connected zone. Intensity indicates that the measurement is used to grow a region from a seed point and to segment it. As each unallocated nearby pixel in the area is compared, the region's size increases. To compute similarity, the difference between the intensity value of a pixel and the region's mean is used. The pixel is assigned to the area, and the minor difference is calculated. The operation is terminated when the intensity difference between the region means and the new pixel exceeds a predetermined threshold. Each pixel's intensity values are compared to those of its neighbors starting with the seed, and if they are within the threshold, the pixel is labeled as one [219]. Next, an image of a tumor-bearing lung is uploaded. The growth's starting point (pixel) coordinate is established, and the base value stores the selected point's color intensity. Next, the initial pixel is stored in an array's coordinates. The process continues until all pixels are eligible and the queue is full. The tumor tissue refers to all pixels in the points array that create a surface. The outermost pixels are also introduced as the tumor boundary, which is curved [224].

Table 7 shows the pros and cons of segmentation methods.

## 7. Feature Extraction

Feature extraction is a process that reduces an initial collection of raw data into more manageable groups that are easier to process [228]. It reduces the number of features in a dataset by creating new ones from existing ones. The feature extraction strategy provides new features that directly blend with the existing elements. When compared to the first feature esteems, the new arrangement of elements will have various qualities [229]. The main point is that fewer features will be required to capture comparable data [230].

### 7.1. Type of Features

Some features need to be extracted and selected to detect lung nodules and cancer more efficiently. There are three kinds of features. If these features are removed, the outcome can be boosted.

#### 7.1.1. Shape-Based Feature

Shape features are significant because they give an option in contrast to depicting an object, utilizing its many attributes, and diminishing how much data are put away. It is one of the most fundamental characteristics of a mass. The irregularity of the mass's shape makes removal difficult [231]. It is classified into two types: region-based techniques and contour-based techniques. A curve estimation method, peak point characterization, and peak line following calculation are all used. Local procedures use the entire item region for its shape highlights, while form-based techniques use data in an article. Shape highlights are classifications of a morphological part.  Figure 5 shows the shape-based features very clearly.

The article "A Comprehensive Survey on the Progress, Process, and Challenges of Lung Cancer Detection and Classification" was published in 2022. Journal: J Healthc Eng.

#### 7.1.2. Texture-Based Feature

The texture is used to segment pictures into areas of interest and group those locales. It refers to all spatial area variations and the selection of general visual perfection or harshness of images. The texture is defined as the spatial distribution of force levels in a given area. They provide invaluable information about the underlying object arrangements of action in a picture, as well as their relationship to climate [231]. Texture-based features are shown in Figure 6.

#### 7.1.3. Intensity-Based Feature

Intensity refers to how much light is emitted or the mathematical worth of a pixel. As demonstrated by image feature intensity, it first requests insights that rely upon individual pixel esteems. The intensity of the light varies from pixel to pixel [231]. Therefore, pixel intensity is the most easily accessible pattern recognition component. Shading is typically addressed by three or four-part intensities in a shading imaging system. The mode, median, standard deviation, and variance of image intensity can all be used to evaluate it.  Figure 7 gives a clear view of intensity-based features.

### 7.2. Feature Extraction Methods

The feature extraction strategy gives us new elements, which are considered a straight mix of the current features. The new arrangement of features will have various qualities when contrasted with the first feature esteems. The fundamental point is that fewer features will be needed to catch similar data.

#### 7.2.1. Radiomics

Radiomics is a strategy that separates an enormous number of provisions from clinical pictures utilizing information portrayal measurements [232]. Radiomic highlights may reveal growth examples and qualities that the unaided eye does not recognize [233]. The standard radiomic investigation includes the evaluation of size, shape, and textural highlights that contain useful spatial data on pixel or voxel circulation and examples [234]. Echegaray et al. [235], Vial et al. [236], and Pankaj et al. [237] used the radiomics method for feature extraction. Mahon et al. [238] used radiomic radiology to extract features.

The article "A Comprehensive Survey on the Progress, Process, and Challenges of Lung Cancer Detection and Classification" was published in 2022. Journal: J Healthc Eng.

#### 7.2.2. Transfer Learning and Fine-Tuning

It first trains a base network on a base informational index and undertakes transfer learning. Afterward, it exchanges the learned components to a subsequent objective organization to prepare for objective informational collection and errand. It trains a model on a dataset and uses it for preparing another dataset [239]. Nishio et al. [240], Sajja et al. [159], and da Nóbrega et al. [241] used transfer learning for lung cancer. Haarburger et al. [242], Marentakis et al. [94], Paul et al. [243], and Tan et al. [244] fine-tuned image to extract features. It takes the underlying patterns, and then a pretrained model has learned and adjusted its outputs to be more suited to your problem. It saves preparation time, does better execution of neural organizations, does not require a great deal of data, and can prompt higher exactness.

#### 7.2.3. LSTM + CNN

The LSTM strategy has turned into a fundamental structure square of neural NLP [245]. To strongly approve of moving examples, some use them as contributions to a value-based classification approximate to the first LSTM production [246]. The CNN long short-term memory network, or CNN LSTM for short, is LSTM engineering explicitly intended for grouping expectation issues with spatial information sources, similar to pictures or recordings. Concerning the improvement of the CNN LSTM model design for system expectations. Tekade and Rajeswari [247] used a layer of CNN LSTM for feature extraction in lung image datasets. Pictures can also be addressed with high-request statistical features processed from run-length matrices or frequent models. Statistics are basic measurements that help us for better comprehension of our pictures [248].

#### 7.2.4. Standard Deviation

Standard deviation limits the ratio of reserves or dispersions of many properties. A low-quality deviation indicates that the properties will be close to the set average as a general rule. In contrast, an elite requirement deviation suggests that the properties will cover a large area [249].

(5) $$\begin{array}{c} \sigma =\sqrt{\frac{1}{N}\overset{N}{\underset{i=1}{\sum }}{\left(S_{i}-\mu \right)}^{2}}\text{,} \end{array}$$

where *σ* is the population standard deviation, *N* means the size of items, *S*_*i*_ is each value from the set, and *µ* is the mean of all the values.

#### 7.2.5. Variance

Variance is the inconstancy in the model expectation—how much the ML capacity can change contingent upon the given informational collection [250]. In this technique, the modified term quantifies how far each number is from the mean and how far each unit number is from the mean [251].

(6) $$\begin{array}{c} \overset{n-1}{\underset{i=0}{\sum }}\overset{n-1}{\underset{j=0}{\sum }}{\left(i-\mu \right)}^{2}\cdot p\left(i,j\right)\;, \end{array}$$

where *µ* is the mean of all the values.

The article "A Comprehensive Survey on the Progress, Process, and Challenges of Lung Cancer Detection and Classification" was published in 2022. Journal: J Healthc Eng.

#### 7.2.6. Mean

Mean is a method for executing feature extraction. It ascertains and takes away the mean for each component. A typical practice is similar to separate this worth by the reach or standard deviation.

(7) $$\begin{array}{c} \mu =\frac{1}{N}\overset{N}{\underset{i=1}{\sum }}S_{i}\text{,} \end{array}$$

where *σ* is the population standard deviation, *N* is the total amount of pixel present in the segmented region, *S*_*i*_ is each value from the set, and *µ* is the mean of all the values.

#### 7.2.7. Fourth-Moment Kurtosis

The kurtosis *k* is characterized to be the normalized fourth focal second. The fourth second is kurtosis, which indicates the level of focal “peakedness” or, more accurately, the “largeness” of the external tails. Kurtosis denotes whether the data have been significantly or lightly followed by the traditional course [252].

(8) $$\begin{array}{c} ku={\left(\frac{1}{N*\sigma^{4}}*\overset{N}{\underset{i=1}{\sum }}\;{\left(S_{i}-\mu \right)}^{4}\right)}^{1/4}\text{,} \end{array}$$

where *σ* is the population standard deviation, *N* is the total amount of pixel present in the segmented region, *S*_*i*_ is each value from the set, and *µ* is the mean of all the values.

#### 7.2.8. Third-Moment Skewness

Skewness is a proportion of the evenness of a circulation. It estimates the measure of likelihood in the tails [253]. The worth is frequently compared to the kurtosis of the average conveyance, which is equal to three. If the kurtosis is more remarkable than three, the dataset has heavier tails than a typical appropriation [254].

(9) $$\begin{array}{c} sk={\left(\frac{1}{N*\theta }*\overset{N}{\underset{i=1}{\sum }}\;{\left(s_{i}-\mu \right)}^{3}\right)}^{1/3}\text{,} \end{array}$$

where *σ* is the population standard deviation, *N* is the total amount of pixel present in the segmented region, *S*_*i*_ is each value from the set, and *µ* is the mean of all the values.

#### 7.2.9. Entropy

Entropy is a substantial proportion of irregularity that can describe the surface of the info picture. In image processing, discrete entropy is a proportion of the number of pieces needed to encode picture data [255]. It distinguishes different communication signals by describing the signals' distribution state characteristics. It is utilized in any course of weight assurance. It is vigorous and computationally fundamental. The higher the entropy value is, the more detailed the image will be. Entropy is a proportion of haphazardness or confusion and thus a proportion of vulnerability [256]. Hussain et al. [257] used entropy to analyze lung cancer image data.

(10) $$\begin{array}{c} \overset{n-1}{\underset{i,j=0}{\sum }}-\ln\;\left(P_{ij}\right)P_{ij}\text{.} \end{array}$$

The article "A Comprehensive Survey on the Progress, Process, and Challenges of Lung Cancer Detection and Classification" was published in 2022. Journal: J Healthc Eng.

#### 7.2.10. Autoencoders

Autoencoder is a sort of neural network that is utilized to gain proficiency with a compacted portrayal of unrefined information [258]. An autoencoder is made up of an encoder and a decoder submodel [259]. The encoder compresses the information, and the decoder attempts to reproduce the contribution from the encoder's compressed variant. Ahmed et al. [260], Z. Wang and Y. Wang [261], Z. Wang and Y. Wang [262], and Kumar et al. [22] used an autoencoder to extract the feature and classify lung nodules. The encoder compresses the input lung scan, and the decoder attempts to recreate the input lung scan from the compressed version provided by the encoder. It can be incredible to highlight extraction, conservativeness, and speed in using backpropagation.

#### 7.2.11. Wavelet

Wavelet is a frequency-selective modulation technique [263]. The wavelet change can assist with changing over the sign into a structure that makes it a lot simpler for our pinnacle locator work. Sometime after the first ECG signal, the wave coefficient for each scale is plotted. Wavelet was used by Kumar et al. [22] to extract features. Soufi et al. [264] attempted to detect lung cancer using a wavelet. Park et al. [265] included and extracted a large number of wavelet features. A discrete wavelet transform (DWT) decomposes a signal into sets of numbers. Every set is a period series of coefficients portraying the time development of the signal in the corresponding frequency band (DWT). DWT is an effective tool for multiresolution analysis, and it is primarily pursued in signal processing, image analysis, and various classification systems [266]. It is broadly used in feature extraction as it is efficient, which can be declared by seeing its previous results.

#### 7.2.12. Histogram of Oriented Gradients (HOG) Features

HOG, or histogram of oriented gradients, is a feature extractor that is frequently used to extract features from picture information [266]. Adetiba and Olugbara [267] used HOG to improve image clarity. Xie et al. [268] used a variety of feature extraction methods, including HOG. Firmino et al. [269] used HOG to extract features from lung image data to detect cancer.

(i) Mathematically, for a given vector *V*:
  (11) $$\begin{array}{c} V=\left[a1,a2,a3,\ldots .,a36\right]\text{.} \end{array}$$
(ii) We calculate root of the sum of squares:
  (12) $$\begin{array}{c} k=\sqrt{{\left(a1\right)}^{2}+{\left(a2\right)}^{2}+{\left(a3\right)}^{2}+\ldots +{\left(a36\right)}^{2}}\text{.} \end{array}$$
(iii) Divide all the values in the vector *V* with this value (*K*):
  (13) $$\begin{array}{c} normalized\;vector=\left(\frac{a_{1}}{k},\frac{a_{2}}{k},\frac{a_{3}}{k},\ldots ,\frac{a_{36}}{k}\right)\text{.} \end{array}$$

The article "A Comprehensive Survey on the Progress, Process, and Challenges of Lung Cancer Detection and Classification" was published in 2022. Journal: J Healthc Eng.

#### 7.2.13. AlexNet, VGG16, and VGG19

AlexNet is the name of a CNN that usually affects AI in a way that unequivocally selects some way of looking at a machine [270]. It joined ReLU initiation after each convolutional and completely associated layer. VGG16 is a CNN model that is represented in the paper by Zisserman from the University of Oxford in their survey [271]. The model achieved 92.7% of the top-5 test accuracy on ImageNet (a dataset of fourteen million + images, including one thousand classes). The most striking feature of the VGG16 is that, unlike many other hyperboundaries, it consistently empties the convolution layers and uses the same cushioning and max pool [272]. VGG19 is a 19-level deep vascular neural entity. Creating more than 1,000,000 images from the Imagine information base can save an organization's pretrained presentation. Khan et al. [273] presented a pretrained VGG19-based automated segmentation and classification technique for analyzing lung CT images that achieved 97.83% accuracy.

Table 8 shows the pros and cons of feature extraction methods.

## 8. Feature Selection

Feature selection refers to reducing the number of input variables required to develop a predictive model. It would be preferable to reduce the number of input variables that can lower the overall computing cost of the model and, in some cases, improve its performance [281]. The primary advantage of feature selection is that it aids in determining the significance of the original feature set.

### 8.1. Genetic Algorithm (GA)

GA is used to identify the most relevant features for lung nodule detection. The GA generates a binary chromosome of 4096 bits in length evaluated offline during the CADe system's training phase.

Logic “1” indicates that this feature is relevant, and logic “0” means irrelevant. As a result, it is removed from the test phase's optimized feature vector. The fitness function is then calculated for each of the population's chromosomes [282]. It uses an evolutionary approach to determine an efficient set from lung images. The initial stage in feature selection is to create a population based on subsets of the possible characteristics derived through lung feature extraction. Then, the subsets of this population are evaluated using a predictive model for the target task.

The article "A Comprehensive Survey on the Progress, Process, and Challenges of Lung Cancer Detection and Classification" was published in 2022. Journal: J Healthc Eng.

### 8.2. mRMR

The minimum redundancy maximum relevance (mRMR) [93] algorithm is a filtering approach that attempts to minimize repetition between selected characteristics while also choosing the most linked attributes with class tags. First, the method determines a collection of features from lung images that have the highest correlation with the class (output) and the lowest correlation among themselves [283]. Then, it ranks features based on mutual information using the minimal-redundancy maximal-relevance criterion. Finally, a measure is used to eliminate redundancy between features, which is stated as follows:

(14) $$\begin{array}{c} mRMR\;\left(F_{j}\right)=\max_{F_{j}\in F\setminus S}\left[I\left(F_{j};C_{k}\right)\right.\\ -\frac{1}{m-1}\underset{F_{i}\in S}{\sum }I\left(F_{j};F_{i}\right)\text{,} \end{array}$$

where *I*(*F*_*j*_;*C*_*k*_) represents the mutual correlation between feature *X*_*j*_ and class *C*_*k*_, *I*(*F*_*j*_;*F*_*i*_) represents the correlation between features *F*_*i*_ and *F*_*j*_, *S* denotes the selected feature set, and *m* means its size (i.e., *m* = |*S*|).

### 8.3. Least Absolute Shrinkage and Selection Operator (LASSO)

The LASSO [284] is a method for modeling the relationship between one or more explanatory factors and a dependent variable by fitting a regularized least-squares model to the dependent variable. It can efficiently identify significant characteristics related to the dependent variable from a small number of observations with many features when used for compressed sensing. For example, it uses lung data by regularizing and selecting the most significant features simultaneously.

### 8.4. Sequential Floating Forward Selection (SFFS)

The SFFS is a bottom-up search procedure that starts with the current feature set and adds new features by applying the basic SFS procedure. Then, if there is still room for improvement in the previous set, the worst feature in the new set is removed. It counts the number of backward steps taken after each forward step [285]. If an intermediate solution at the fundamental level cannot be improved upon, there are no backward steps. The procedure's inverse counterpart, on the other hand, can be described similarly. Because both algorithms provide “self-controlled backtracking,” it is possible to find practical solutions by dynamically modifying the trade-off between forwarding and backward steps. They analyze what they require in a way that does not rely on any parameters [286]. To begin, it starts with an empty set. Then, SFFS takes backward steps on lung images after each step as long as the objective function increases. It reduces the number of unnecessary features from lung images.

The article "A Comprehensive Survey on the Progress, Process, and Challenges of Lung Cancer Detection and Classification" was published in 2022. Journal: J Healthc Eng.

### 8.5. PCA

PCA is a dimensionality-reduction approach commonly used to reduce the dimensionality of data by lowering an extensive collection of variables into a smaller set of variables that retains the majority of the learning from the large set of variables [287]. In addition, smaller datasets are easier to analyze and visualize, making them more accessible. For example, it chooses characteristics from lung images based on the magnitude of their coefficients.

### 8.6. Weight Optimized Neural Networks with Maximum Likelihood Boosting (WONN-MLB)

Newton and Raphson's MLMR preprocessing model and the boosted weighted optimized neural network ensemble classification algorithms are used to develop the WONN-MLB [288]. The additive combination approach is utilized in the WONN-MLB method to incorporate the highest relevancy with the least amount of redundancy. To achieve the goal of lung cancer detection accuracy with the least amount of time and error, an ensemble of WONN-MLB qualities is used [289]. It only overviewed the extracted features from the lung feature based on the probability.

### 8.7. Hybrid Intelligent Spiral Optimization-Based Generalized Rough Set Approach (HSOGR)

The hybrid intelligent spiral optimization-based generalized rough set approach (HSOGR) [90] is used to select the features. The spiral optimization method [290] is based on spiral phenomena and aids in the resolution of the unconstrained optimization problem when picking features. The approach employs adequate settings such as convergence and periodic descent direction in the *n*-dimensional spiral model to achieve success. The approach predicts optimization characteristics according to the exploration (global solution) and exploitation (local key) phases with the help of the parameters (good solution). Rather than using a single gradient function when selecting an optimization process, this method employs several spiral points [291], which aid in the establishment of the current optimal fact at any given time. To determine whether the selected characteristics accurately aid in detecting lung cancer, the search space must be investigated using a generalized rough set procedure.

Table 9 shows the pros and cons of feature selection methods.

## 9. Classification and Detection

A classification algorithm is an algorithm that gauges the information included, so the yield isolates one class into positive qualities and the other into negative qualities [297]. The classification methodology is a supervised learning strategy used to recognize classes of novel perceptions based on information preparation [298].

The article "A Comprehensive Survey on the Progress, Process, and Challenges of Lung Cancer Detection and Classification" was published in 2022. Journal: J Healthc Eng.

Detection is a computer innovation connected with computer vision and image processing that arranges with recognizing occasions of semantic objects of a specific class in computerized pictures and recordings [299]. It is a computer vision strategy for finding objects in pictures or recordings. When humans look at pictures or videos, objects can be perceived and found in minutes. The objective of object detection is to reproduce this intelligence utilizing a computer [68]. In addition, well-informed areas of article recognition incorporate face location and passerby identification.

### 9.1. Machine Learning (ML)

Machine learning is a subordinate part of artificial intelligence, which is comprehensively characterized as the ability of a machine to impersonate shrewd human conduct [300]. This implies machines that can perceive a visual scene, comprehend a text written in ordinary language, or play out an activity in the actual world [301]. In addition, machine learning calculations utilize computational techniques to “learn” data straightforwardly from information without depending on a foreordained condition as a model [302].  Table 10 describes various types of machine learning (ML) algorithms.

### 9.2. Deep Learning (DL)

DL is a subfield of ML and AI that copies the path of individual achieving knowledge [313]. Deep learning uses both organized and disorganized information, like text and images, to train the models [314]. Deep learning methods are stored in a sequential pattern for complexity and abstraction, whereas established ML methods are linear [315]. Moreover, deep learning eliminates some data preprocessing techniques and can extract features automatically [316]. Several deep methods have gained tremendous results. They are described in Table 11.

### 9.3. Convolutional Neural Network (CNN)

A convolutional neural network (CNN) is a methodology under DL that is capable of taking in input images, emphasizing different objects from the image, and distinguishing continuously [329]. In addition, CNNs are considered a type of neural network that allows for more feature extraction from captured images [330]. CNNs are classified into three categories: convolution, max-pooling, and activation [331]. In comparison to other classifiers, a CNN requires little preprocessing. Although the filters are hand-engineered in a primitive way, CNN can learn these filters/features through adequate training [332].  Table 12 describes the usage of CNN to detect lung nodules and cancer.

### 9.4. Hybrid System

A hybrid structure of CNN with LeNet and AlexNet is developed for analysis by combining the layer settings of LeNet with the parameter settings of AlexNet. It begins with the LeNet architecture, incorporates ReLU, LRN, and dropout layers into the framework, and finally develops the Agile CNN. In addition to two fully connected layers, the proposed CNN, based on LeNet, has two convolutional layers, two pooling layers, and two fully connected layers. Layer C1 contains 20 feature maps for each feature map in total. The input data for each unit are linked to a neighborhood. Therefore, a connection from the input cannot extend outside the confines of the feature map boundary. The first feature map in P1 is connected to the second feature map in C1 by 22 neighborhoods. Every unit in P1 is linked to the second feature map in C1. Then, on layer C2, there are 50 feature maps. The other options are the same as they were for the previous layers. F1 and F2 are the final two layers after layer P2. In terms of neuron units, F1 and F2 have 500 and 2 neuron units, respectively. The effect of the parameters of the kernel size, learning rate, and other aspects on the performance of the CNN model is explored by varying these parameters, and an optimized setup of the CNN model is obtained as a result [339]. There are various hybrid methods to detect lung cancer and nodules [340–343].  Figure 8 gives an overview of CNN's hybrid structure. In artificial intelligence, the image is commonly convolved with a particular filter (HOG or LBP) to enhance shapes and edges. Consequently, the first stage of CNN consists primarily of Gabor-like filters. Additionally, the scale-space method was initially designed to enhance the CNN method on which we based. We proposed a novel hybrid CNN model by incorporating standard features into CNN, considering complementary characteristics of the conventional texture method and CNN. This hybrid model's complex distinguishable higher-level features are made up of one-of-a-kind combinations of low-level features. The CNN filters have this hierarchy of simple elements to complex features: the first layer filters mostly have structures that look like Gabor. In contrast, the deep layer filters in the network have features that can be identified as objects. In this study, we combine CNN with texture features like LBP and HOG to improve the first layer filters, which are analogous to the human visual system's ability to decompose images into their oriented spatial frequencies. The data input layer, convolution layer, pooling layer, entire connection layer, and output layer are typically included in the structure of a CNN network. By combining data, our hybrid CNN model aims to make the data input layer easier. In contrast, the primary objective of the training is to discover the optimal model parameters by minimizing a loss function. It has been found that HOG features and LBP features are fused with CNN in a specific way due to the significant differences in shape and texture between the benign and malignant nodules. However, CNN is believed to be able to extract lung nodules with possible distinguishing features.

The article "A Comprehensive Survey on the Progress, Process, and Challenges of Lung Cancer Detection and Classification" was published in 2022. Journal: J Healthc Eng.

### 9.5. Transfer Learning

Transfer learning refers to a methodology wherein the put-away information came about. Learning a model while settling a particular errand can address alternate undertaking of a related issue. Deep convolutional neural networks have accomplished amazing feats in normal picture examination. In any case, such incredible feats are exceptionally subject to the dataset. Transfer learning is a difficult substitute for examining nodules in clinical images using DCNN models, with the only aim of regulating deep CNN terrifying exposure due to the limited amount of clinical images. Some authors used transfer learning in their research [155, 159, 240, 241, 303, 309, 344, 345]. The basic framework of transfer learning is shown in Figure 9.

## 10. Performance Evaluation

It is hard to choose which metrics to use for various issues, and observational studies have shown yet assessed graphic elements to gauge different parts of the calculations [346]. It is often difficult to say which measurements are most appropriate for evaluating the analysis due to the frequent weight gain errors between the expected and actual values [347]. The interpretation of ML estimations is reviewed depending upon critical accuracy, which is routinely improper, assuming that there ought to emerge an occurrence of unequaled information and error cost shift strikingly [175]. ML execution evaluations include a degree of compromise between the true positive and accurate negative rate and between recall and precision. The receiver operating characteristic (ROC) curve depicts the compromise between the false negative and false positive rates for each possible cutoff.

### 10.1. Generally Used Evaluation Metrics

Evaluation metrics are considered a way of quantifying the effectiveness of a predictive model. Evaluation metrics are used to ensure the quality of a statistical or ML model. When evaluating your model, it is essential to use a variety of different evaluation metrics [348].

- True positive (TP): TP is the correct classification of the positive class. For instance, if an image contains destructive cells and the model fragments the diseased part effectively, the result classifies cancer.
- True negative (TN): TN is the correct classification of the negative class, for example, when there is no malignant growth in the image. The model after classification declares that the cancer is absent.
- False positive (FP): FP is the erroneous prediction of the positives; for instance, the picture has carcinogenic cells, but the model classifies that the image does not contain cancer.
- False negative (FN): FN is the false expectation of the negatives. For instance, there is no malignancy in the picture except for the model that says an image is a carcinogenic one [349].

The article "A Comprehensive Survey on the Progress, Process, and Challenges of Lung Cancer Detection and Classification" was published in 2022. Journal: J Healthc Eng.

The effectiveness of any ML model is still up in the air utilizing measures like TP rate, FP rate, TN rate, and FN rate [350]. The sensitivity and specificity measures are commonly used to clarify demonstrative clinical tests as well as to assess how excellent and predictable the diagnostic test is [37]. The TP rate or positive class accuracy is the sensitivity measurement, while the TN rate or negative class accuracy refers to the specificity measurement [351]. There is frequently a compromise between the four measurements in “real-world” applications.

### 10.2. Classification Measurements

There are a lot of methods used for the classification of lung nodule and lung cancer. The widely used metrics for classification problems are as follows.

#### 10.2.1. Precision

Precision is the number of relevant reports recovered by a search isolated by the number of pieces retrieved. In short, precision is the number of pieces recovered that are important. It checks how exactly the model functions by actually taking a look at the correct, true positives from the anticipated ones [249].

(15) $$\begin{array}{c} Prec.=\frac{TP}{TP+FN}\text{.} \end{array}$$

#### 10.2.2. Recall/Sensitivity

Recall/sensitivity is the number of pertinent records recovered by a search isolated by existing significant archives. Sensitivity is another name for recall. The test's sensitivity reflects the likelihood that the screening test will be positive among unhealthy people. The number of applicable archives recovered is referred to as recall. It computes the number of true positives detected by the model and marks them as positives [352]. Finally, it estimates the capacity of a test to be positive when the condition is present. It is otherwise called false negative rate, review, Type II error, *β* error, error or oversight, or elective theory [69].

(16) $$\begin{array}{c} Recall=\frac{TP}{TP+FN}\text{.} \end{array}$$

#### 10.2.3. Accuracy

Accuracy is the level of closeness to ground truth. For example, the accuracy of an estimation is a proportion of how close the deliberate worth is to the actual value of the amount. The estimation accuracy might rely upon a few factors, including the breaking point or the goal of the estimating instrument [353].

(17) $$\begin{array}{c} Accuracy=\frac{TP+TN}{TP+TN+FP+FN}\text{,} \end{array}$$

where TP, TN, FP, and FN mean true positive, true negative, false positive, and false positive, respectively.

The article "A Comprehensive Survey on the Progress, Process, and Challenges of Lung Cancer Detection and Classification" was published in 2022. Journal: J Healthc Eng.

Aside from this, there are other types of accuracy, such as predictive accuracy and average accuracy. Predictive accuracy should be estimated based on the difference between observed and predicted values [354, 355]. Average accuracy is the average of every accuracy per class (amount of accuracy for each class anticipated/number of classes) [356].

#### 10.2.4. F1-Score

*F*-Measure or F1-score combines both precision and recall into a binary measure that catches the two properties, giving each similar weighting. The arithmetic mean of the two proportions is precision and recall [357]. The *F*-measure is used to fine-tune precision and recall. It is frequently used for evaluating data recovery frameworks, such as search engines, as well as some types of ML models, particularly in natural language processing [358]. F1-score is the function of precision and recall. It is evaluated when a balance between precision and recall is needed [359].

(18) $$\begin{array}{c} F1=\frac{precision\times recall\;}{precision+recall\;}\text{.} \end{array}$$

#### 10.2.5. Specificity

Specificity is the capacity of a test to distinguish individuals without illness effectively. The test's specificity reflects the likelihood that the screening test will be negative among people who do not have the illness. It estimates a test's ability to be harmful when the condition is not present. It is otherwise called FP rate, precision, Type I error, *α* error, error of commission, or null hypothesis [278].

(19) $$\begin{array}{c} Specificity=\frac{TN}{TN+FP}\text{.} \end{array}$$

#### 10.2.6. Receiver Operating Characteristic Curve (ROC Curve) and Area under the ROC Curve (AUC)

A ROC curve is a graphical plot that outlines the symptomatic capacity of a twofold classifier framework as its separation edge is fluctuated [360]. ROC analysis provides methods for selecting ideal models and automatically removing imperfect ones from the expense setting or class conveyance. ROC analysis is directly and naturally linked to cost/benefit analysis of demonstrative dynamics [361]. ROC curves are considered a fantastic asset as an accurate display measure in location/characterization hypothesis and speculation testing. For a variety of reasons, AUC is often preferred over accuracy [362]. Indeed, since it is probably the most widely used performance metric, it is very uncomfortable to adjust how AUC works [363] properly.

#### 10.2.7. ROC Curve

The ROC curve addresses the performance of the proposed model at all characterization limits [364]. The ROC curve summarizes classifier execution over a range of TP and FP error rates. It is a graph of the true positive rate versus the false positive rate (TPR versus FPR). A point on the ROC curve between (0, 100) would be ideal [365]. ROC helps investigate the compromises among various classifiers over a scope of situations, which is not great for circumstances with realized error costs [366–369].

(20) $$\begin{array}{c} TPR=\frac{TP}{TP+FN}\text{,}\\ FPR=\frac{FP}{FP+TN}\text{.} \end{array}$$

The article "A Comprehensive Survey on the Progress, Process, and Challenges of Lung Cancer Detection and Classification" was published in 2022. Journal: J Healthc Eng.

#### 10.2.8. AUC

AUC coordinates the region under the ROC curve from (0, 0) to (1, 1). It gives the total proportion of all conceivable characterization edges [370]. AUC has a range of 0 to 1. The AUC esteem for a correctly classified version will be 1.0, while it will be 0.0 in the case of a completely incorrect classification [371]. It is amazing for two reasons: first, it is scale-invariant, which means it examines how well the model is anticipated rather than the overall qualities; and second, it is grouping limit invariant, which means it examines the model's exhibition regardless of the chosen edge [372]. The region under the curve (AUC) is most favored because the bigger the region, the better the model. The AUC additionally has a decent translation as the likelihood that the classifier positions an arbitrarily picked positive occasion over a haphazardly picked negative one [373]. The AUC is a useful measurement for classifier execution because it is independent of the chosen standard and earlier probabilities [374]. AUC can be used to establish a predominance connection between classifiers. If the ROC curves cross, the absolute AUC is a normal comparison between models [375–380].

### 10.3. Segmentation Measurements

There are a lot of methods used for the segmentation of lung nodule and lung cancer. The widely used metrics for segmentation problems are as follows.

### 10.4. Jaccard Index

The Jaccard index, otherwise called the Jaccard similarity coefficient, is a measurement that checks the closeness and variety of test sets. It is defined as the width of the crossing point divided by the width of the association of two name sets. It is a proportion of comparability for the two information arrangements, ranging from 0% to 100% [382]. The higher the rate, the more comparable the two populaces.

(21) $$\begin{array}{c} {Jac}_{idx}=\frac{TP}{TP+FP+FN}\text{.} \end{array}$$

### 10.5. Dice Coefficient

The Dice similarity coefficient, otherwise called the Sorensen–Dice list or Dice coefficient, is a factual instrument that estimates the comparability between two arrangements of information [383]. The Dice coefficient should not be more noteworthy than 1. A Dice coefficient, for the most part, goes from 0 to 1 [384]. If the coefficient result is greater than 1, the execution may need to be rechecked [385]. It was used as a measurable approval metric to evaluate the reproducibility of manual divisions as well as the spatial crossover precision of robotized probabilistic partial division of MR images, as represented on two clinical models [386–388]. It is a substantial proportion of the comparability rate between two example sets:

(22) $$\begin{array}{c} {Dice}^{cof}=\frac{2\times TP}{2\times TP+FP+FN}\text{.} \end{array}$$

The article "A Comprehensive Survey on the Progress, Process, and Challenges of Lung Cancer Detection and Classification" was published in 2022. Journal: J Healthc Eng.

### 10.6. Error Calculation

The term “error” refers to a deviation from accuracy or correctness. Errors are considered a significant issue when anyone wants to evaluate the system's performance. When the performance is evaluated, only the system's efficiency is calculated. But the errors must be measured while calculating the performance. Many techniques are available to calculate the errors in lung cancer detection.

#### 10.6.1. Mean Absolute Error (MAE)

MAE is a model assessment metric utilized with relapse models. The mean outright error regarding a test set is the mean of the absolute values of the individual prediction errors on all examples in the test set. In insights, MAE is a proportion of errors between combined perceptions communicating a similar wonder [389, 390].

(23) $$\begin{array}{c} MAE=\frac{\left|p_{1}-a_{1}\right|+\ldots +\left|p_{n}-a_{n}\right|}{n}\text{,} \end{array}$$

where *p* represents predicted target values (*p*_1_, *p*_2_,…, *p*_*n*_) while *a* represents actual value: *a*_1_, *a*_2_, ..., *a*_*n*_, in which *n* represents total number of data points.

#### 10.6.2. Root Mean Square Error (RMSE)

RMSE is the square root of the mean of the square of the entirety of the error. RMSE is a good proportion of accuracy, but it should only be used to analyze and compare prediction errors of different models or model setups for a single variable, not between factors because it is scale-dependent [249].

(24) $$\begin{array}{c} RMSE=\sqrt{\frac{{\left(p_{1}-a_{1}\right)}^{2}+\ldots +{\left(p_{n}-a_{n}\right)}^{2}}{n}}\text{,} \end{array}$$

where *p* represents predicted target values (*p*_1_, *p*_2_,…, *p*_*n*_) while *a* represents actual value: *a*_1_, *a*_2_,…, *a*_*n*_, in which *n* represents total number of data points.

#### 10.6.3. Relative Absolute Error

RAE is a way of estimating the performance of a proactive model. RAE is a metric contrasting genuine figure error with the estimated error of a shortsighted (naive) model. A sensible model (which produces results that are superior to a trivial model) will bring about a proportion short of one [391, 392].

The article "A Comprehensive Survey on the Progress, Process, and Challenges of Lung Cancer Detection and Classification" was published in 2022. Journal: J Healthc Eng.

#### 10.6.4. Root Relative Squared Error (RRSE)

The RRSE is comparable with what it would have been if a straightforward indicator had been utilized. To put it bluntly, this specific indicator is only the average of the actual values. In this way, the relative squared error standardizes the total squared error by partitioning it by the absolute squared error of the forward indicators. By taking the square root of the relative squared error, one decreases the error to similar measurements as the amount being anticipated [393, 394].

(25) $$\begin{array}{c} \sqrt{\frac{{\left(p_{1}-\bar{a}\right)}^{2}+\ldots +{\left(p_{n}-a_{n}\right)}^{2}}{{\left|a_{1}-\bar{a}\right|}^{2}+\ldots +{\left|a_{n}-\bar{a}\right|}^{2}}}\text{,} \end{array}$$

where *p* represents predicted target values (*p*_1_, *p*_2_,…, *p*_*n*_) while *a* represents actual value: *a*_1_, *a*_2_,…, *a*_*n*_.

## 11. Challenges and Research Direction

Lung cancer detection techniques are improving day by day. Currently, available lung cancer detection techniques are quite good in terms of performance, but there are many more limitations that researchers have encountered. Many issues have been resolved, but some remain.

Some of them are mentioned below.

### 11.1. Insufficient Number of Annotated Medical Datasets with Cases

Most of the significant successes of deep learning techniques in general, and convolutional neural networks in particular, have been achieved using large amounts of data. Large annotated datasets of lung CT images are in high demand, but obtaining such datasets in medical imaging remains challenging due to various factors, such as the time-consuming nature of clinician annotation tasks, the need for privacy, and ethical considerations, among others. Expert radiologists must construct and annotate large datasets, which is costly and time consuming. As a result, the insufficiency of datasets with a large number of samples is a significant barrier to the application of deep learning to the study of medical data [17].

### 11.2. Accurate Segmentation

Accurate segmentation of the lung fields is necessary to efficiently reduce the search space for lung nodules. Due to inhomogeneities within the lung region and similar density pulmonary components such as arteries, veins, bronchi, and bronchioles, technical issues concerning lung segmentation techniques should be researched further. These technical difficulties include the technique's automation level, sensitivity to scanning parameters, an algorithm's ability to work with multiple image modalities (e.g., CT, LDCT, or CE-CT), and the algorithm's ability to provide proper lung segmentation.

The article "A Comprehensive Survey on the Progress, Process, and Challenges of Lung Cancer Detection and Classification" was published in 2022. Journal: J Healthc Eng.

### 11.3. Nodule Types

Most nodules are harmless, indicating a more severe health issue. Among other tissues, parenchymal tissues are distinct and difficult to segment. On the other hand, solitary and large solid nodules are easy for segmentation. But the problem occurs when these types of nodules are targeted.

#### 11.3.1. Small Nodules

Small-nodule segmentation is critical for the early identification of lung cancer [395]. Thin-slice high-resolution computed tomography (HRCT) has enabled the visibility of tiny nodules less than 5 mm in diameter, which was previously invisible using previous-generation CT technology. Accurate segmentation of such small nodules is required to assess the malignancy of the lesions. A partial-volume effect is the primary technical concern when dealing with tiny nodules (PVE). The spatial discrimination used in CT imaging allows a single voxel to represent multiple tissue types by averaging their intensity values. This induces PVE and picture blur, particularly near lesion margins, challenging segmentation. When dealing with smaller lesions, PVE becomes more pronounced since the fraction of mistakes over the lesion volume increases. This makes measuring the area/volume of tiny nodules more difficult. The partial-volume approach (PVM) [396] is presented for calculating nodule volume based on the consistency of the average attenuation quantities. PVM outperforms other thresholding algorithms in volumetric accuracy, according to their phantom study. SPVA (segmentation-based partial-volume analysis) [397] is proposed to extend the PVM approach to include VOI segmentation into the nodule core, parenchyma area, and partial-volume region. A histogram from the partial volume region was used to estimate the volume of the nodule near its boundary. Finally, the proposed RAGF [398] yields an elliptical approximation of the lesion boundary.

#### 11.3.2. Nodules Attached to Vessels

Lung nodules are frequently connected to other pulmonary structures such as the airways, blood vessels, parenchymal walls, and diaphragm. Because the CT values of nodules and these non-target objects are frequently extremely similar, determining the extent of the nodule from these structures becomes a difficult technical issue. Juxta-vascular nodules are nodules that connect to blood vessels. Morphological filtering is a systematic strategy for this purpose [397, 399–403]. Because the proportion of nodules that attach to vessels/airways is often minimal compared to the entire extent of the 3D nodule surface, basic MOs such as erosion, dilatation, and opening are frequently effective in most juxta-vascular situations [400, 402]. These fundamental operators were combined with convex-hull operations [397, 404] and 3D moment analysis [405] to refine the segmentation process after it was completed. Geometric/shape constrained segmentation is another prominent strategy in this context [398, 403, 406–408]. This method incorporates shape-based prior information into the segmentation process to bias the results toward a spherical/nodular shape. It suppresses elongated non-target components linked to the target.

The article "A Comprehensive Survey on the Progress, Process, and Challenges of Lung Cancer Detection and Classification" was published in 2022. Journal: J Healthc Eng.

#### 11.3.3. Nodules Attached to Parenchymal Wall and Diaphragm

Juxta-pleural nodules are cases that are attached to the parenchymal wall or the diaphragm. These nodules are connected to the chest wall and pleural surface. Many automated measurement algorithms struggle with these nodules because they need to determine where the nodule ends and the chest wall begins. Solitary nodules, on the other hand, that do not border any other structures, such as airways or blood arteries, are much easier to segment [409].

#### 11.3.4. Ground-Glass Opacity Nodules

The ground-glass opacity (GGO) nodule is a nodule with subsolid CT values that are much lower than usual solid nodules. They are classified into two types based on whether or not solid components are present: non-solid/pure and partially solid/mixed. GGO nodule segmentation is a technological issue because it is difficult to distinguish their tiny boundaries and model their uneven appearances. In clinical practice, modern CT technology's more excellent picture resolution has enabled the investigation of small GGO nodules. Although their growth is frequently slow [410], such GGO nodules, particularly mixed ones, have been linked to a high risk of malignancy [411]. Recent clinical studies are part of the histological spectrum of peripheral adenocarcinomas, which encompass premalignant atypical adenomatous hyperplasia (AAH) and malignant bronchioloalveolar carcinoma (BAC) [412]. Over ten years, a tiny non-solid GGO representing AAH or BAC can gradually grow into an invasive lung adenocarcinoma [410]. In this method, segmentation is accomplished by labeling each voxel with a nodule/background label based on a probabilistic decision rule established from training data.

### 11.4. Article Selection Bias

A measurement of association, such as a risk ratio, that is distorted as a result of sample selection that does not accurately reflect the target population is known as selection bias. The selection of individuals, groups, or data for analysis in such a way that proper randomization is not achieved, failing to ensure that the obtained sample is representative of the intended population, is known as selection bias. On the other hand, selection bias might be an issue: the sociodemographic profile of DLCST participants was better. They had greater psychological fortitude than the general population of people who smoked a lot [413]. As a result, selection bias could lead to underestimating the actual psychosocial effects [413]. According to a psychometric analysis of survey data and qualitative focus group interviews, abnormal and false positive LCS results can have a wide range of psychosocial effects that can be adequately quantified with PROMs [414, 415]. The finest articles and specifics of each are described in Table 13.

The article "A Comprehensive Survey on the Progress, Process, and Challenges of Lung Cancer Detection and Classification" was published in 2022. Journal: J Healthc Eng.

### 11.5. Efficient CADe System

Developing an efficient computer-aided detection (CADe) system for detecting lung nodules is a difficult task. The level of automation, speed, and ability to recognize nodules of varying shapes, such as irregularly shaped nodules rather than only spherical ones, as well as the CADe system's ability to detect cavity nodules, nodules attached to the lung borders, and small nodules, are all critical considerations to consider (e.g., less than 3 mm).

### 11.6. Volumetric Measurements

Volumetric measurements are essential because various sizes in different situations make the system more accurate. When calculating the growth rate in the volumetric unit, the global movement of patients caused by their actions and the local activity of the entire lung tissue caused by respiration and heartbeat should be considered. It is impossible to distinguish between changes caused by the direct application of global and local registration to the segmented nodule and changes in the shape of the nodule caused by breathing and heartbeat.

The research directions that should be inspected to uplift the lung nodule and cancer detection outcomes are described here. Through profound investigation on this topic, the recommendations for the study are described below.

Table 14 represents challenges and limitations in lung nodule and cancer diagnosis, as well as research directions in terms of the dataset, architectures, and so on.

- Datasets focused on CT scans are available openly. Ultrasound, PET scans, and SPECT datasets, on the other hand, are not publicly available. Furthermore, studies utilizing such imaging modalities use unpublished datasets. These datasets should be made public for future research and implementations.
- Like U-Net and SegNet, segmentation models have provided sophisticated segmentation results across various image datasets. Furthermore, implementing these techniques involving different modalities may improve lung nodule and cancer detection results.
- All kinds of nodules need to be investigated. Implementing feature extraction and selection can detect any nodule. The selection of features and classifiers can be used to identify nodules. The most common methods for selecting features are genetic algorithms, WONN-MLB, and HSOGR. Feature extraction, on the other hand, is critical for detecting nodules. Most of the time, radiomic methods extract features from lung images. HOG, autoencoders, and wavelets should also be investigated to be more accurate.
- Random forest, SVM, DBN with RM, and CNNs are primarily used for lung cancer diagnosis. ML techniques such as boosting, decision trees, and DL networks of various types such as GANs and clustering should be analyzed. CNN is widely used to detect lung nodules and cancer because it can extract essential features from images. CNN can identify and classify lung cancer types with greater accuracy in a shorter period. But as CNN is a DL model, it needs a massive amount of data, so if the dataset is insufficient, it will not give benchmark accuracy. We recommend that strategies based on different CNN architectures and CNN+ and other dimensional CNN must be inquired.
- When patients are breathing, their lung shape changes, and it varies from patient to patient. The patient's lung cancer cells appeared in large numbers, and there were more irregular shapes than in healthy lungs. Availability of all datasets is needed to measure all kinds of lungs. We recommend investigating all datasets and measuring different shapes of lungs. The authors in [419, 420] have already started working on this idea.

The article "A Comprehensive Survey on the Progress, Process, and Challenges of Lung Cancer Detection and Classification" was published in 2022. Journal: J Healthc Eng.

## 12. Conclusions

Lung cancer is the most widely recognized disease-related reason for death among people. Early detection of pulmonary nodules and lung cancer saves lives because it is known that the chances of surviving cancer are higher if it is found, diagnosed, and treated quickly. Several methods and systems have been proposed for analyzing pulmonary nodules in medical images. Additionally, the domain covers biological, engineering, computer science, and histological research. However, this article provides a comprehensive overview of the lung cancer detection interface. It is intended for novices interested in learning about the present state of lung cancer detection methods and technologies. The essential concepts of lung cancer detection methods are fully explored. The article focuses on many aspects of the research domain, including image preprocessing, feature extraction, segmentation, feature selection methodologies, performance measurements, and challenges and limitations along with the possible solutions. The article endorses a summary of current methods to help new researchers quickly understand the research domain conceptions. The study also looks into the various types of datasets available to lung cancer detection systems. The fundamental principles of lung cancer detection and nodule classification procedures are thoroughly explored using CT scan, MRI, or X-ray imaging. Furthermore, the article combines current cancer-detecting systems, describing a preliminary review based on previous works. The article also describes the challenges and limitations that will help explore the inconvenience of lung cancer detection technologies. The majority of lung cancer detection methods are now in the primary stages of development. Still, there are many things that could be changed to make the system work better. The combined efforts of scientific researchers and the tech sectors are required to commercialize this vast area for the benefit of ordinary people.

The article "A Comprehensive Survey on the Progress, Process, and Challenges of Lung Cancer Detection and Classification" was published in 2022. Journal: J Healthc Eng.

## Figures and Tables

**Figure 1:** The workflow diagram of basic CAD system.

**Figure 2:** A taxonomy of AI-based lung nodule and cancer diagnosis.

**Figure 3:** The PRISMA process that is followed in this article.

**Figure 4:** Word cloud of the title and selected articles on lung cancer.

**Figure 5:** Shape-based features.

**Figure 6:** Texture-based features.

**Figure 7:** Intensity-based features.

**Figure 8:** Brief overview of hybrid structure of CNN. Each yellow box is to train the machine with data, blue boxes have layers and parameters for individual machines, and purple boxes have layers for one to nth hybrid models.

**Figure 9:** Basic structure of transfer learning.

**Table 1:** A comparison of different surveys based on lung nodules and cancer detection.

Survey			Ref	[27]	[28]	[29]	[30]	[31]	[32]	[33]	[34]	[35]	Ours
			Year	2018	2019	2019	2020	2020	2020	2020	2021	2021	—
Taxonomy				✗	✗	✗	✗	✗	✗	✓	✗	✗	✓
Dataset				✓	✓	✓	✓	✓	✓	✓	✓	✓	✓
Image preprocessing				✓	✗	✗	✗	✓	✗	✓	✓	✗	✓
Feature extraction				✗	✗	✗	✓	✓	✓	✓	✓	✓	✓
Segmentation				✓	✓	✓	✓	✓	✓	✓	✓	✓	✓
Feature selection				✓	✗	✗	✗	✗	✗	✗	✓	✓	✓
Image modalities				✗	✓	✗	✓	✗	✓	✗	✓	✗	✓
Evaluation metrics				✗	✓	✓	✓	✓	✓	✗	✓	✗	✓
Challenges				✗	✓	✓	✗	✓	✗	✗	✗	✗	✓
AI based	Machine learning			✗	✓	✓	✓	✗	✓	✓	✓	✓	✓
	Deep learning	CNN		✗	✗	✗	✓	✗	✗	✗	✗	✗	✓
		Other		✓	✗	✗	✗	✓	✓	✓	✓	✓	✓

**Table 2:** A summary of recent surveys/reviews on various lung cancer detection, segmentation, and classification techniques.

Ref.	Purposes	Challenges
[36]	Deep learning techniques are used to detect, segment, and classify pulmonary nodules in CT scans	Generalization ability problem for learning-based methods. It happens because of the different training datasets and the methods.
[29]	A comprehensive analysis of deep learning with convolutional neural network (CNN) methods and their performances	Problems with the generalizability and explication of the detection results, lack of accurate clinical decision-making tools, and well-labeled medical datasets
[30]	The review of recent studies in lung nodule detection and classification provides an insight into technological advancements	Low sensitivity, high false positive rate, time-consuming, small database, poor performance rates, and so on
[4]	A comparison of various machine learning-based methods for detecting lung cancer has been presented	Mainly focuses on machine learning techniques for classification rather than other processes. Also avoid the MRI type data.
[31]	Review of recent deep learning algorithms and architectures for lung cancer detection	The data and the unbalanced nature of it are the current limitations
[37]	Discussing the most recent developments in the field	The size of the target object within the image makes it difficult to implement a CNN; as the size of the target object varies, studies proposed training the model with images of varying scales to teach the model about this size variation
[38]	Providing an accurate diagnosis and prognosis is essential in lung cancer treatment selection and planning	Incorporating knowledge from clinical and biological studies into deep learning methods and utilizing and integrating multiple medical imaging methods
[27]	Algorithms used for each processing step are presented for some of the most current state-of-the-art CAD systems	Limitation of more interactive systems that allow for better use of automated methods in CT scan analysis
[33]	An overview of the current state-of-the-art deep learning-aided lung cancer detection methods, as well as their key concepts and focus areas	Limited datasets and high correlation of errors in handling large image sizes
[35]	A summary of existing CAD approaches for preprocessing, lung segmentation, false positive reduction, lung nodule detection, segmentation, classification, and retrieval using deep learning on CT scan data	Deficient data annotation, overfitting, lack of interpretability, and uncertainty quantification (UQ)
[39]	A survey of what CADe schemes are used to detect pulmonary nodules will help radiologists make better diagnoses	Slight increase in lung density and micronodules whose diameters are less than 3 mm are difficult to detect. For multimodality, clinical records and medical images are not combined.

The article "A Comprehensive Survey on the Progress, Process, and Challenges of Lung Cancer Detection and Classification" was published in 2022. Journal: J Healthc Eng.

**Table 3:** The criteria used to choose which review articles to include and which ones to exclude.

Inclusion/exclusion	Criteria
Inclusion	IC1: English language is used to write research papers
	IC2: all papers related to the lung cancer detection process
	IC3: publications in academic journals, book chapters, conference/workshop proceedings, and thesis dissertations
	IC4: published articles between the years 2000 and 2022 (in the survey, a few old papers are used for a specific purpose)
	IC5: articles being available with full text

Exclusion	EC1: not fitting with the theme of the review
	EC2: duplicate articles
	EC3: low-quality papers
	EC4: lack of enough information
	EC5: full text not available

**Table 4:** Different types of datasets of lung.

Dataset name	Image type	Used in	Unit	Link
LIDC-IDRI	CT scan images	[7, 19, 22, 23, 31, 42–60]	1018	[61]
LUNA16	CT scan (which was gathered from LIDC-IDRI with slice thickness less than 3 mm)	[18, 19, 42, 44, 49, 57, 60, 62–84]	888	[15]
NSLT	Low-dose CT images and chest radiographs	[85, 86]	3410	[87]
The Cancer Imaging Archive (TCIA)	All kind of CT scan and X-ray	[50, 88–96]	3.3 million images	[97]
Society of Radiological Technology (JSRT)	X-ray	[98–102]	154	[100]

**Table 5:** Advantages and disadvantages of imaging modality methods.

Methods	Advantages	Disadvantages
X-ray	Harmlessly and easily helps to analyze sickness and screen treatment	It can harm cells in the body, which thus can build the danger of creating malignant growth. CT scan is better than X-ray.
CT scan	It is easy, painless, and precise. It has the capacity to picture bone, delicate tissue, and veins all simultaneously. It gives point-by-point pictures of many kinds of tissue.	It requires breath holding and radiation which is difficult for a few patients
Magnetic resonance imaging (MRI)	It does not include radiation and is more averse to deliver an unfavorably susceptible response that might happen when iodine-based substances are utilized for X-beams and CT checks	The time required for an MRI is longer than CT. Additionally, MRI is typically less inclined to be quickly accessible than CT.
Positron emission tomography (PET) scan	It diminishes the quantity of examining meetings a patient should go through	Slow developing, less dynamic cancers may not assimilate a lot of tracer
Single-photon emission computed tomography (SPECT)	It tends to be seen in various planes and to isolate covering structures	It has significant expense and less accessibility

**Table 6:** Advantages and disadvantages of image preprocessing methods.

Algorithms	Advantages	Disadvantages
Histogram equalization [190]	It is a versatile strategy to the picture and an invertible administrator. It can be recuperated and expands differentiation of pictures.	It is not the best technique for contrast improvement and is unpredictable. It expands the contrast of foundation noise.
Median filter mask [10]	It can save sharp components in a picture while filtering noise, and it is good at eliminating “salt and pepper” type noise	It separates picture edges and produces false noise edges and cannot smooth medium-tailed noise dissemination
Gaussian filter [191]	Its Fourier change has zero recurrence. It is broadly utilized to diminish picture noise and lessen detail.	It decreases subtleties and cannot deal with “salt and pepper” noise. It sometimes makes all parts blue and obscures the objects.
Wiener filter [192]	It eliminates the additive noise, transforms the obscuring, and limits the general mean square error during inverse filtering and noise smoothing	It is hard to acquire ideal rebuilding for the noise, relatively delayed to apply as working in the recurrence area
Gabor filter [151]	It investigates whether there is a particular recurrence content. It has gotten significant consideration as it takes after the human visual framework.	It requires huge investments. It has a high excess of provisions.
Isotropic voxel [193]	It is the fastest approach and a “precise” 3D structure block, as it copies particles and opens new reproduction procedures	It is hard to fabricate complex articles utilizing voxels. It does not have numerical accuracy.
Thresholding [142]	It diminishes the intricacy, works on acknowledgment and grouping, and changes the pixels to make the picture simpler	There is no assurance that the pixels distinguished by the thresholding system are bordering
Binary inversion [194]	CT scans were converted into black and white to detect the nodules as binary inversion will get the dark part as black which means 1	It is not a clear form to detect nodules and it has a huge chance to miss the nodules
Interpolation [195]	It is used to foresee obscure qualities. It forecasts values for cubic in a raster.	It obscures the edges when the decreased proportion is less
SMOTE [179]	It is an oversampling procedure and is powerful to handle class awkwardness. It assists with conquering the overfitting issue.	It can build the covering of classes and present extra commotion. Often it does not constrict the predisposition.
CLAHE [187]	The adjoining tiles are joined using bilinear expansion to take out incorrect representation incited bounds	Any commotion that might be accessible in the picture

The article "A Comprehensive Survey on the Progress, Process, and Challenges of Lung Cancer Detection and Classification" was published in 2022. Journal: J Healthc Eng.

**Table 7:** Advantages and disadvantages of segmentation methods.

Algorithms	Advantages	Disadvantages
Watershed [225]	Being able to divide an image into its components	Takes too long to run in order to meet the deadline, sensitivity to false edges and over-segmentation
U-Net [226]	Images can be segmented quickly and accurately	Redundancy occurs due to patch overlap, also relatively slow
MV-CNN [203]	No user-interactive parameters or assumptions about the shape of nodules are needed	The loss of gradients may have an effect
CF-CNN [206]	Gathered sensitive information about nodules from CT imaging data	Less adaptable for small nodules and cavitary nodules
FCM [188]	Ignored noise sensitivity limitation, successfully overcoming the PCM's clustering problem	Row sum constraints must be equal to one in order to work
Hessian-based approaches [209]	High robustness against noise and sensitivity to small objects	Performance decreases for large nodule
SegNet + shape driven level set [213]	Correct seed point initialization with no manual intervention in the level set	Segments the lung nodule partly occluded, also takes a longer time
Faster R-CNN [214]	The efficiency of detection is high	It could take a long time to reach convergence
Mask R-CNN [218]	Easy to train, generalizable to other tasks, effective, and only adds a minor overhead	Low-resolution motion blur detection typically fails to pick up on objects
RASM [219]	Well suited to large shape models and parallel implementation allowing for short computation times	Cannot segment areas with sharp angles and is not built to handle juxta-pleural nodules
Region growing [227]	The concept is simple, multiple criteria can be selected simultaneously, and it performs well in terms of noise	Computing is time-consuming. Noise or variation may result in holes or over-segmentation, making it difficult to distinguish the shading of real images.

**Table 8:** Advantages and disadvantages of feature extraction methods.

Algorithms	Advantages	Disadvantages
Radiomics [274]	It could extricate and distinguish many provisions and component types. It has a minimal expense.	For respiratory movement, it obscures data. It has restricted data of remade pictures.
Transfer learning and fine-tuning [244]	It saves preparation time, does better execution of neural organizations, does not require a great deal of data, and can prompt higher exactness	Transfer learning has the issue of negative exchange. Fine-tuning can at some point befuddle to sort out subclasses.
LSTM + CNN [94]	It is appropriate to separate compelling elements and group, process, and foresee time series given delays of obscure length	It is inclined to overfitting, and it is hard to apply as it requires 4 direct layers which require a lot of memory
Standard deviation [275]	It gives an exact thought of how the data are appropriated. It is detached by outrageous qualities.	It tends to be affected by anomalies, is hard to ascertain or comprehend, and works out all vulnerability as error
Autoencoder [276]	It can be incredible for highlight extraction, conservativeness, and speed in coding utilizing backpropagation	It cannot deal with adequate preparation information, prepares some unacceptable use cases, and is excessively lossy
Variance [277]	It treats all deviations from the mean and assists an association with being proactive in accomplishing targets	It gives added weight to anomalies, is not effectively deciphered, and does not offer wonderful precision
Fourth-moment kurtosis [50]	It will be in the positive structure, and conveyance about the mean gets tighter as the mean gets bigger	The weakness is that it will not have a negative or indistinct structure
Wavelet [278]	It offers a synchronous restriction on schedule and recurrence space. It is quick and can isolate the fine subtleties in a sign.	It has shift affectability, its directionality is poor, and it has absence of stage data
Entropy [279]	It is utilized in any course of weight assurance. It is vigorous and computationally basic.	It has restricted critical thinking part and relative disparity, contingent upon the given length and biasing
Histogram of oriented gradients [267]	It shows invariance to photometric changes by making a dark foundation with white molecules which sharpens the articles unmistakably	The last descriptor vector develops bigger to set more effort to extricate and to prepare utilizing a given classifier
Third-moment skewness [50]	It is smarter to gauge the presentation of the speculation returns, transforming the data point of high skewness into slanted conveyance	It is eccentric. The ascent and defeat of a network are best instances of the skewness.
AlexNet, VGG16, and VGG19 [280]	AlexNet has 8 layers that exceed the yield dissimilar to other enactment capacities. VGG is an incredible structure block for learning reasons.	AlexNet battles to examine all provisions accordingly delivering helpless performing models. VGGNet is agonizing to prepare and its loads itself are very huge.

The article "A Comprehensive Survey on the Progress, Process, and Challenges of Lung Cancer Detection and Classification" was published in 2022. Journal: J Healthc Eng.

**Table 9:** Advantages and disadvantages of feature selection methods.

Algorithms	Advantages	Disadvantages
GA [292]	Tries to avoid becoming stuck in a local optimal solution	GA does not guarantee an optimal solution and has high computational cost
mRMR [293]	Effectively reduces the redundant features while keeping the relevant features	Mutual information is incompatible with continuous data
LASSO [294]	Very accurate prediction, reduces overfitting, and improves model interpretability	In terms of independent risk factors, the regression coefficients may not be consistently interpretable
SFFS [295]	Reduces the number of nesting issues and unnecessary features	Difficult to detect all subsets
PCA [296]	Selects a number of important individuals from all the feature components, reduces the dimensionality of the original samples, and improves the classification accuracy	Only considers the linear relationships and interaction between variables at a higher level
WONN-MLB [288]	Integrates the maximum relevancy and minimum redundancy	Has certain amount of irrelevant attributes
HSOGR [90]	Effectively selects optimized features	Its execution is complex

**Table 10:** Most commonly utilized machine learning classifiers for classifying nodules and cancer.

Model name	Purpose	Data type	Result	Strength	Limitation
RF [303]	Using pretrained model to detect lung cancer accurately	CT	Acc 82.5%	Improves the capacity of lung nodule prediction	Limited dataset and result
SVM [300]	Classifying the lung nodules in four lung cancer stages	CT	Acc 84.58%	Predicts small-sized lung nodules, even in low density	The limited dataset affected their results
LDA [301]	Classifying cancer using ODNN and LDA	CT	Acc 94.56%	It is quick, easy to use, non-invasive, and inexpensive	Optimal feature selection with multiclassifier was missing
RF [304]	Automatic classification of pulmonary peri-fissural nodules (PFNs)	CT	Sens 86.8%	Pretrained CNNs are employed, which makes them faster than training CNNs	All kinds of nodules were not classified
SVM [78]	To increase the accurate prediction of lung cancer	CT	Acc 85.7%	Predicts lung cancer from low-resolution data images	The model sometimes fails to predict
RF [299]	To detect malignancy of nodules with self-built model NoduleX	CT	Pres 99%	Solid, part-solid, and non-solid nodule categorization is performed automatically	Big nodules were accurately detected
RF [305]	Classified the measured solidity or nodules	CT	Acc 95%	Avoids potential errors caused by inaccurate image processing	The description of their work is not described clearly
SVM [306]	An improved FP-reduction method is used to detect lung nodules in PET/CT images	CT	Spec 97.2%	Removes around half of the existing FPs	Only small cohort is used
Boosting [307]	Classification of nodules with fusion of texture, shape, and deep model-learned data	CT	F1 96.65%	Generates more accurate outcomes than three existing state-of-the-art techniques	The model only detects big nodules
Multikernel learning [302]	Distinguishing between the nodule and non-nodule classes with classification	CT	Acc 94.17%	Increases the efficacy of false positive reduction	Dataset name is unclear
SVM [308]	Extracting absolute information inherent in raw hand-crafted imaging components	CT	Acc 95.5%	Obtains promising classification outcomes	The reference is limited
Decision tree [22]	Using autoencoder with decision tree to detect nodule	CT	Sens 75.01%	Outperforms the state-of-the-art techniques on the overall accuracy measure, even after experimenting with nearly five times the data amount	The results are low
SVM [309]	Nodule classification with hybrid features	CT	Acc 99.3%	It extracts the representative image of lung nodule malignancy from chest CT images	The model cannot detect type, position, and size
Decision tree [310]	Discovering radiomics to detect lung cancer	CT	Sens 77.52%	Increases the accuracy of lung cancer prediction diagnostics	The reference is limited and results are low
Boosting [66]	Identifying nodules from CT scan	CT	AUC 86.42%	Quickly finds the exact positions of latent lung nodule	The references of figure and table are accurately done
Multikernel learning [311]	To describe the algorithm for false positive reduction in lung nodule computer-aided detection (CAD)	CT	Jindex 91.39%	Automatically reduces unnecessary feature subsets to get a more discriminative feature set with promising classification performance	All false positive reduction is not done yet
Logistic regression [312]	Prediction of the malignancy of lung nodules in CT scans	CT	Sens 94.5%	Additional information based on nodule size has at best a mixed impact on classifier performance	It only takes large nodules
DBScan [68]	Detecting nodules with 3D DCNN	CT	Spec 79.67%	It can be expanded into other areas of medical image identification	FP reduction and automated classification are missing
Naïve Bayes [243]	A pretrained CNN to extract deep features from lung cancer images and train classifiers to predict all term survivors	CT	Acc 82.5%	The method's performance is such that adding nodule size information has only a mixed effect on classifier performance	The dataset was too small

The article "A Comprehensive Survey on the Progress, Process, and Challenges of Lung Cancer Detection and Classification" was published in 2022. Journal: J Healthc Eng.

**Table 11:** Most commonly utilized deep learning classifiers for classifying nodules and cancer.

Model name	Purpose	Data type	Result (%)	Strength	Limitation
DBN with RBM [317]	To detect nodules with deep networks	CT	Acc 92.83	No relative location information is ignored to extract features that express the original image better	The references were very limited with less info of method
DRL [318]	Detecting lung cancer with several potential deep reinforcement learning models	CT	Acc 80	Got promising results in tumor localization	The result of their work is not fully cleared
DRN [319]	Detecting lung cancer in FDG-PET imaging under ultra-low-dose PET scans	PET	Acc 97.1	Lung cancer detection is automated even at low effective radiation doses	The outcome is insufficient
DBN with RBM [320]	Testing the feasibility of using DL algorithms for lung cancer diagnosis	CT	Acc 79.40	It has shown very promising results	Accuracy was slightly less than CNN model
Deep denoising autoencoder [321]	A combination of deep-learned representations was employed to create a lengthy feature vector, which was then used to train the classification of nodules	CT	Acc 95.5	Increased the ability to differentiate between malignant and benign nodules, with a significant improvement in sensitivity	The dataset was not a benchmarked dataset
DRN [322]	Training model first and applying 3D ConvNet to detect lung nodule with hybrid loss learning	CT	Acc 86.7	It detects pulmonary nodules from low-dose CT scans	Detects small nodules and cannot classify malignant or benign nodules
DBN with RBM [23]	Comparing DL and CNN model on lung nodule detection	CT	Sens 73.4	It solves the longstanding challenge of classifying lung nodules as malignant or benign without computing morphological or textural data	The classification was very limited
DRN [323]	Identification of lung nodules from CT scans is efficient for lung cancer diagnosis, and false positive reduction is important, so it was the aim	CT	Acc 98	It is reliable and detects well. It may also be easily extended to detect 3D objects.	Figures and table are not referred clearly
DRL [77]	Developing and validating a reinforcement learning model for early identification of lung nodules in CT images	CT	Acc 99.1	Eliminated the major issue of false positives in CT lung nodule screening, saving unwanted tests and expenditures	Only the big nodules were detected
Deep denoising autoencoder [324]	A spherical harmonic expansion is used as it has ability to approximate the surfaces of tough shapes of the detected lung nodules	CT	Acc 96	It can show small or big lung nodule spatial inhomogeneities	Classification of nodule as malignant or benign was not done
Multilayer perceptron model [325]	To analyze the performance of several ML methods for detecting lung cancer	CT	Acc 88.55	The presented image preprocessing method detects cancerous bulk	The layers of the model were not discussed briefly
Deep stacked autoencoder [326]	The main purpose is to train a 3D CNN with data and convert it into a 3D fully convolutional network (FCN) that can generate the score map	CT	Sens 80	It can generate the score map for the whole volume in a single pass	The results were not compared with other models
Deep sparse autoencoder [327]	Analyzing the nodules of CT data and helping the experts to be more the accurate with proposed analysis tool	CT	Acc 99.57	Improving the display of actual medical CT data may automatically extract pulmonary nodule features	The information of dataset is missing
GAN [328]	Building a 3D U-Net and CNN to segment and identify nodule and assist the radiologists understand CT images	CT	Acc 95.4	Malignant nodule detection is precise and effective	Detects large nodule more accurately than the small nodules
Deep stacked autoencoder [260]	To get an accurate diagnosis of the detected lung nodules	CT	Acc 92.20	It classified nodules using higher-order MGRF and geometric criteria	They did not mention any reshape or resize techniques

The article "A Comprehensive Survey on the Progress, Process, and Challenges of Lung Cancer Detection and Classification" was published in 2022. Journal: J Healthc Eng.

**Table 12:** Different types of CNN models.

Model name	Purpose	Data type	Result (%)	Strength	Limitation
MV-CNN [54]	Malignant nodule characterization	CT	Acc 92.31	It is a fast and reliable computer-aided system	A large amount of labeled data is needed for better accuracy
MP-CNN [333]	Automatic detection of lung cancer	CT	Acc 87.80, spec, 89.10, recall 87.40	It uses both local and global contextual variables to detect lung cancer	Different image size affects the accuracy
HSCNN [334]	To predict the malignancy of a pulmonary nodule seen on a computed tomography (CT) scan	CT	Acc 84.40, sens 70.50, spec 88.90, AUC 85.60	Model interpretability improves with prediction accuracy	No domain specialists can fine-tune it by prioritizing more discriminating features under challenging cases
NODULEX (CNN features + QIF features) [335]	Differentiate between malignant and benign nodule patterns with accuracy	CT	Acc 94.60, sens, 94.80, spec 94.30	Excellent accuracy in classifying nodule malignancy	Cross-validated results may be less accurate. Other datasets with significantly differing CT scan picture quality or criteria were not directly fit.
DENSEBTNET (centercrop operation) [336]	Identifying multiscale features in nodule candidates	CT	Acc 88.31, AUC 93.25	It has good parameter efficiency and is parameter light. It enhances DenseNet performance and classification accuracy over other approaches.	Its densely connected mechanism causes feature redundancy
PN-SAMP [337]	Accurately identifying the nodule areas, extracting semantic information from the detected nodules, and predicting the malignancy of the nodules	CT	Acc 97.58	It can predict the malignancy of lung nodules and offer high-level semantic features and nodule location	Only works on CT images
Dual-pathway CNN [338]	Predicting the nodule's malignancy	CT	Acc 86.84	It performs end-to-end lung nodule diagnostics with high classification accuracy. It can also handle smaller datasets using transfer learning.	A pulmonary nodule cannot be detected automatically
DeepLung (DUAL-path 3D DCNN+) [71]	Developing a fully automated lung CT cancer detection system	CT	Acc 90.44	It is smaller and more efficient than residual networks	Lung nodule annotation is not satisfactory
Ensemble learning of CNNS/multiview knowledge-based collaboration (MV-KBC) [268]	Differentiating between malignant and benign pulmonary nodules	CT	Acc 91.60, AUC 95.70	It uses an adaptive weighting system learned during error backpropagation to categorize lung nodules, allowing the MV-KBC model to be trained end-to-end	During training, there is a relatively high level of computational complexity

The article "A Comprehensive Survey on the Progress, Process, and Challenges of Lung Cancer Detection and Classification" was published in 2022. Journal: J Healthc Eng.

**Table 13:** Best articles and their details.

Author info	Patient group	Outcomes	Key results	Comments
Raz et al. [417](USA) (retrospective cohort study (level 4, good))	37 patients identified with isolated adrenal metastases from NSCLC	5-year survival	34% in the adrenalectomy group versus 0% in the non-operative group (*P*=0.002)	The selection process for operative and non-operative management was inconsistent
	20 underwent surgical resection		83% for ipsilateral tumors versus 0% for contralateral tumors (*P*=0.003)	Adrenalectomy patients were on average 10 years younger
	17 underwent non-operative management		67% in case of lower lobe NSCLC versus 27% in cases of upper lobe tumors (*P*=0.29)	50% of patients in the adrenalectomy group (and 70% in the non-operated group) had N2 or T4 diseases; therefore, the adrenal metastasis was not truly isolated
	Maximum follow-up period of 16 years		27% synchronous metastasis versus 41% metachronous metastases (*P*=0.81)	Significant variability in treatment with chemotherapy and radiotherapy
			52% with N0 or N1 disease versus 0% with N2 diseases (*P*=0.008)	

Luketich and Burt [418] (USA) (retrospective cohort study (level 4, good))	14 patients with isolated synchronous adrenal metastasis from NSCLC	Medium survival	Medium survival of 8.5 months in the chemotherapy alone group versus 31 months in the chemotherapy + surgery group	Small study, but no significant differences were seen in preoperative characteristics, tumor size, or cell type to otherwise explain the improved survival
	8 patients had neoadjuvant chemotherapy followed by concomitant lung resection and adrenalectomy		In the surgically resected group, the 3-year actuarial survival was 38%	
	6 patients had only 3 cycles of chemotherapy (mitomycin, cisplatin, and vinblastine)		Longest survivor at end of follow-up was 61 months	The authors recommend that surgery should be advocated after ensuring that curative resection of the lung primary can be achieved
	5-year follow-up			

Higashiyama et al. [416] (retrospective cohort study (level 4, good))	9 patients with isolated adrenal metastases from surgically resected lung cancer (4 non-curative and 5 curative)	Survival	Adrenalectomy group: 2/5 alive at 24 and 40 months, respectively, and 3/5 died at 9, 17, and 20 months, respectively	All patients in the palliative group had a disease-free interval of 7 months. This selection bias may explain some of the observed difference in survival in addition to the influence of treatment strategy.
	5 treated with adrenalectomy followed by adjuvant chemo or radiotherapy			
	4 treated with palliative chemo or radiotherapy		Palliative group: all died within 6 months	The authors concluded that short FDIs are probably due to lymphatic spread and probably signify a more aggressive tumor
	Maximum follow-up of 40 months			

The article "A Comprehensive Survey on the Progress, Process, and Challenges of Lung Cancer Detection and Classification" was published in 2022. Journal: J Healthc Eng.

**Table 14:** Challenges and research directions for lung nodule and cancer diagnosis.

Name	Challenges	Research direction
Insufficient number of annotated medical datasets with cases	All datasets are not publicly available	All datasets need to be available openly. Additionally, research should be conducted utilizing such imaging modalities using unpublished datasets. All datasets should be disclosed for future research works and implementations.
Accurate segmentation	Segmentation models are not properly executed	All segmentation models need to be implementing in various modalities which may uplift the lung nodule and cancer detection results
Nodule size and types	Small nodules are needed to be detected more efficiently	All kinds of nodules need to be investigated. Implementing feature extraction and selection can detect most of the nodules. Nodules can be identified by feature and classifier selection.
Efficient CADe system	Nodules and cancer detection need to be more accurate using all architectures	Random forest, SVM, DBN with RM, and CNNs are mostly used for lung cancer diagnosis. ML and DL networks of other kinds should be analyzed in this field.
Volumetric measurements	All lung image shapes are not the same. So, all datasets need to be extracted.	When patients are breathing, their lung shape changes and it varies from patient to patient. We recommend investigating all datasets and measuring different shapes of lungs.

## Data Availability

No data were used to support this study.
